# COVID-19 mRNA Vaccines: Lessons Learned from the Registrational Trials and Global Vaccination Campaign

**DOI:** 10.7759/cureus.52876

**Published:** 2024-01-24

**Authors:** M. Nathaniel Mead, Stephanie Seneff, Russ Wolfinger, Jessica Rose, Kris Denhaerynck, Steve Kirsch, Peter A McCullough

**Affiliations:** 1 Biology and Nutritional Epidemiology, Independent Research, Copper Hill, USA; 2 Computer Science and Artificial Intelligence Laboratory, Massachusetts Institute of Technology, Cambridge, USA; 3 Biostatistics and Epidemiology, Independent Research, Research Triangle Park, USA; 4 Immunology and Public Health Research, Independent Research, Ottawa, CAN; 5 Epidemiology and Biostatistics, Independent Research, Basel, CHE; 6 Data Science, Independent Research, Los Angeles, USA; 7 Cardiology, Epidemiology, and Public Health, McCullough Foundation, Dallas, USA; 8 Cardiology, Epidemiology, and Public Health, Truth for Health Foundation, Tucson, USA

**Keywords:** sars-cov-2 (severe acute respiratory syndrome coronavirus -2), risk-benefit assessment, cardiovascular, autoimmune, mortality, gene therapy products, serious adverse events, immunity, registrational trials, covid-19 mrna vaccines

## Abstract

Our understanding of COVID-19 vaccinations and their impact on health and mortality has evolved substantially since the first vaccine rollouts. Published reports from the original randomized phase 3 trials concluded that the COVID-19 mRNA vaccines could greatly reduce COVID-19 symptoms. In the interim, problems with the methods, execution, and reporting of these pivotal trials have emerged. Re-analysis of the Pfizer trial data identified statistically significant increases in serious adverse events (SAEs) in the vaccine group. Numerous SAEs were identified following the Emergency Use Authorization (EUA), including death, cancer, cardiac events, and various autoimmune, hematological, reproductive, and neurological disorders. Furthermore, these products never underwent adequate safety and toxicological testing in accordance with previously established scientific standards. Among the other major topics addressed in this narrative review are the published analyses of serious harms to humans, quality control issues and process-related impurities, mechanisms underlying adverse events (AEs), the immunologic basis for vaccine inefficacy, and concerning mortality trends based on the registrational trial data. The risk-benefit imbalance substantiated by the evidence to date contraindicates further booster injections and suggests that, at a minimum, the mRNA injections should be removed from the childhood immunization program until proper safety and toxicological studies are conducted. Federal agency approval of the COVID-19 mRNA vaccines on a blanket-coverage population-wide basis had no support from an honest assessment of all relevant registrational data and commensurate consideration of risks versus benefits. Given the extensive, well-documented SAEs and unacceptably high harm-to-reward ratio, we urge governments to endorse a global moratorium on the modified mRNA products until all relevant questions pertaining to causality, residual DNA, and aberrant protein production are answered.

## Introduction and background

Our understanding of coronavirus disease 2019 (COVID-19) mRNA vaccinations and their impact on mortality has evolved substantially since the first vaccine rollouts in December 2020. Early investigations indicated the potential of these biologicals for preventing severe acute respiratory syndrome coronavirus 2 (SARS-CoV-2) infection. Based on the first randomized controlled trials sponsored by Pfizer-BioNTech ((New York, United States (US); Mainz, Germany) and Moderna Inc. (Massachusetts, US), researchers concluded that there was a noteworthy 95% relative risk (RR) reduction of symptomatic COVID-19 [1,2]. The overlapping finding between the two trials prompted the US Food and Drug Administration (FDA) to allow the use of the COVID-19 mRNA vaccines under Emergency Use Authorization (EUA) on December 11, 2020, a decision that was followed by early unblinding and cessation of the trials [3].

Prior to the rapid authorization process, no vaccine had been permitted for market release without undergoing a testing period of at least four years, the record set by Merck & Co., Inc. (New Jersey, US) in 1967 with the development of the world’s first mumps vaccine [4]. Pfizer’s vaccine (BNT162b2) completed the process in seven months. Previous timeframes for phase 3 trial testing averaged 10 years [5]. Health departments have stated that 10-15 years is the normal timeframe for evaluating vaccine safety [6]. With the COVID-19 vaccines, safety was never assessed in a manner commensurate with previously established scientific standards, as numerous safety testing and toxicology protocols typically followed by the FDA were sidestepped [7,8]. Preclinical studies of the mRNA product’s biodistribution and potential toxicities from repeated doses (to mimic multiple vaccinations), were circumvented to enable accelerated clinical testing [9]. Perhaps the most important trial benchmark obviated by the rapid authorization process was the minimum 6-12 month observation period typically recommended for identifying possible longer-term vaccine-related adverse effects (AEs) in the vaccine versus placebo groups [9].

The previously established 10-15-year timeframe for clinical evaluation of vaccines was deemed necessary to ensure adequate time for monitoring the development of AEs such as cancers and autoimmune disorders [10,11]. To be expeditious, the coordinators of Pfizer and Moderna trials prioritized symptomatic COVID-19 risk reduction over severe AEs and mortality concerns. In retrospect, this was a grave misstep. Historical accounts bear witness to instances where vaccines were prematurely introduced to the market under immense pressure, only to reveal disabling or even fatal AEs later on. Examples include the 1955 contamination of polio vaccines, instances of Guillain-Barré syndrome observed in flu vaccine recipients in 1976, and the connection between narcolepsy and a specific flu vaccine in 2009 [12-14]. Against this backdrop, it is not surprising that so many medical and public health experts voiced concerns about the COVID-19 mRNA vaccines bypassing the normal safety testing process [15-17].

Political and financial incentives may have played a key role in undermining the scientific evaluation process leading up to the EUA. Lalani and colleagues documented the major investments made by the US government well before authorization [18]. Even prior to the pandemic, the US National Institutes of Health invested $116 million (35%) in mRNA vaccine technology, the Biomedical Advanced Research and Development Authority (BARDA) had invested $148 million (44%), while the Department of Defense (DOD) contributed $72 million (21%) to mRNA vaccine development. BARDA and the DOD also collaborated closely in the co-development of Moderna’s mRNA vaccine, dedicating over $18 billion, which included guaranteed vaccine purchases [18]. This entailed pre-purchasing hundreds of millions of mRNA vaccine doses, alongside direct financial support for the clinical trials and the expansion of Moderna’s manufacturing capabilities. The public funding provided for developing these products through Operation Warp Speed surpassed investments in any prior public initiative [19]. Once the pandemic began, $29.2 billion (92% of which came from US public funds) was dedicated to the purchase of COVID-19 mRNA products; another $2.2 billion (7%) was channelled into supporting clinical trials, and $108 million (less than 1%) was allocated for manufacturing and basic research [18]. This profuse spending of taxpayer dollars continued throughout the pandemic: BARDA spent another $40 billion in 2021 alone [20].

Using US taxpayer money to purchase so many doses in advance would suggest that, prior to the EUA process, US federal agencies were strongly biased toward successful outcomes for the registrational trials. Moreover, it is reasonable to surmise that such extensive vested interests could have influenced the decision to prematurely halt the registrational trials. Unblinding essentially nullified the “placebo-controlled” element of the trials, eliminating the control group and thus undermining the ability to objectively assess the mRNA vaccines’ safety profile and potential serious AEs (SAEs). Thus, while the accelerated authorization showcased the government’s dedication to provide these novel products, it also raised concerns among many experts regarding risk-benefit issues and effectively eliminated the opportunity to learn about the potential long-range harms of the mRNA inoculations. The political pressures to rapidly deliver a solution may have compromised the thoroughness and integrity of the scientific evaluation process while downplaying and obfuscating scientific concerns about the potential risks associated with mRNA technology.

Concerns about inadequate safety testing extend beyond the usual regulatory approval standards and practices. Although we employ the terms "vaccine" and "vaccination" throughout this paper, the COVID-19 mRNA products are also accurately termed gene therapy products (GTPs) because, in essence, this was a case of GTP technology being applied to vaccination [21]. European regulations mandate the inclusion of an antigen in vaccines, but these immunogenic proteins are not intrinsic to the mRNA vaccines [22]. The GTP vaccine platform has been studied for over 30 years as an experimental cancer treatment, with the terms gene therapy and mRNA vaccination often used interchangeably [23]. This is due to the mRNA products’ specific mode of action: synthetic mRNA strands, encapsulated within a protective lipid nanoparticle (LNP) vehicle, are translated within the cells into a specific protein that subsequently stimulates the immune system against a specific disease. Another accurate label would be prodrugs because these products stimulate the recipient’s body to manufacture the target protein [24]. As there were no specific regulations at the time of the rapid approval process, regulatory agencies quickly “adapted” the products, generalized the definition of “vaccine” to accommodate them, and then authorized them for EUA for the first time ever against a viral disease. However, the rationale for regulating these products as vaccines and excluding them from regulatory oversight as GTPs lacks both scientific and ethical justification [21]. (Note: Throughout this review, the terms vaccines and vaccinations will be used interchangeably with injections, inoculations, biologicals, or simply, products.)

Due to the GTPs’ reclassification as vaccines, none of their components have been thoroughly evaluated for safety. The main concern, in a nutshell, is that the COVID-19 mRNA products may transform body cells into viral protein factories that have no off-switch (i.e., no built-in mechanism to stop or regulate such proliferation), with the spike protein (S-protein) being generated for prolonged periods, causing chronic, systemic inflammation and immune dysfunction [25,26]. This S-protein is the common denominator between the coronavirus and the vaccine, which helps to explain the frequent overlap in AEs generated by both the infection and the inoculation [25]. The vaccine-induced S-protein is more immunogenic than its viral counterpart; and yet, the increased antibody production is also associated with more severe immunopathology and other adverse effects [27]. The Pfizer and Moderna mRNA products contain mRNA with two modified codons that result in a version of the S-protein that is stabilized in its prefusion state [28]. This nucleoside-modified messenger RNA technology is intended to extend the synthetic mRNA’s persistence in the body. When the S-protein enters the bloodstream and disseminates systemically, it may become a contributing factor to diverse AEs in susceptible individuals [25].

In this narrative review, we revisit the registrational trials and review analyses of the AEs from these trials and other relevant studies. Most of the revelations have only recently come to light, due to the past few years of extensive censorship of healthcare professionals and research scientists who challenged the prevailing narrative set forth by the vaccine enterprise [29,30]. We begin with a focus on the two randomized double-blind placebo-controlled trials that resulted in the EUA, followed by an in-depth exploration of the various adverse impacts of the mRNA inoculations, with frequent reference to the original trials. In a post-pandemic context in which the immediate urgency has subsided, exploratory narrative reviews such as this can play an important role in helping us reevaluate the scientific basis for the general public’s well-founded safety concerns regarding the COVID-19 mRNA vaccinations.

## Review

Revisiting the registrational trials

Early in the pandemic, US public health officials promised that the phase 3 trials would prove the COVID-19 mRNA vaccines were “safe and effective”, including a reduction in severe disease, hospitalization, and death, with a secondary endpoint of preventing transmission and infection [31]. Nine vaccine manufacturers issued an unprecedented joint statement pledging not to prematurely seek regulatory review [32]. Both sets of assurances were delivered to a population already suffering from pandemic fatigue, mostly attributable to lockdowns, masking, social distancing, and other restrictions imposed by the same agencies responsible for ushering in the vaccination program. Despite the rhetoric, no large randomized double-blind placebo-controlled trials have ever demonstrated reductions in SARS-CoV-2 transmission, hospitalization, or death.

Importantly, the study designs for the pivotal trials that led to the EUA were never intended to determine whether the mRNA inoculations could help prevent severe disease or premature death [31]. This was mainly due to insufficient statistical power for assessing these outcomes [33]. (The power calculation was based solely on the reduction of COVID-19 symptoms, the primary outcome.) The limitation stemmed from the recruitment of young, healthy trial participants in the 18-55-year age group and the relatively low number of reported clinical infection cases in the intervention arms of the trials, with only eight cases in Pfizer and 11 in Moderna [1,2]. Whereas Pfizer’s trial recorded just one instance of severe COVID-19, Moderna’s trial reported none, leading the company to proclaim 100% efficacy against severe illness [34]. Moderna also reported one COVID-19 death, in the placebo group [2]. Thus, between the two trials, there was only one death attributed to COVID-19 among the more than 73,000 trial participants [1,2].

After announcing the trial’s results, Pfizer extended its study by four months. Trial participants were unblinded by week 20, and placebo volunteers were invited to receive the mRNA vaccination. Pfizer’s announcement of the efficacy of its mRNA product was based on 162 out of 22,000 placebo recipients contracting COVID-19, compared to only eight out of 22,000 vaccine recipients. None of the 162 placebo recipients who contracted COVID-19 died from the disease [35]. These numbers are too small to draw meaningful, pragmatic, or broad-sweeping conclusions with regard to COVID-19 morbidity and mortality [36].

Moreover, the 170 polymerase chain reaction (PCR)-confirmed case count diverts attention from another finding: a much larger number of cases identified during the study fell under the category of “suspected COVID-19,” where individuals exhibited symptomatic COVID-19 but lacked a positive PCR test [37]. (Note: The PCR tests used in these trials were those widely accepted for detecting SARS-CoV-2 and ostensibly met certain standards of performance and reliability for accurate detection of the coronavirus.) A total of 3,410 cases of suspected, unconfirmed COVID-19 were identified, a 20-fold difference between suspected and confirmed cases. There were 1,594 such cases in the vaccinated group, and 1,816 in the placebo. When factoring in both confirmed and suspected cases, vaccine efficacy against developing symptoms drops to only 19%, far below the 50% RR reduction threshold required for regulatory authorization [37]. Even when removing cases occurring within seven days of vaccination to account for short-term vaccine reactogenicity (rather than true infections), efficacy would be a meager 29%. Any false negatives among the suspected cases would tend to further diminish the benefit. Thus, when considering both confirmed and suspected cases, vaccine efficacy appears to have been dramatically lower than the official 95% claim.

Similarly, it is important to emphasize that the “cases” being counted in the trials were PCR-positive patients with mild infections, not moderate to severe illnesses. Thus, a cough or other mild respiratory symptoms qualified as primary endpoints [38,39]. The trial’s conclusion was predicated on a mere 100 of such COVID-19 “cases” recorded within the placebo group [31]. Once the trial reached this point, it was anticipated that efficacy would be declared, and participants in the placebo group would be offered the active vaccine. This was the precise scenario that transpired, with Pfizer’s blinded phase concluding at two months and Moderna’s ending at three, effectively terminating the blinded randomized follow-up period and greatly limiting any risk-benefit evaluations.

The lack of ability to evaluate severe illness in the trials reflected the real-world context, namely that the likelihood of severe COVID-19, hospitalization, and dying from the infection has always been very low. Stratifying by age, the infection fatality rate (IFR) in 2021 showed an age gradient with approximately a three to four-fold increase for each decade, starting as low as 0.0003% (nearly zero) among children and adolescents, increasing to 0.5% in those aged 60-69 [40]. Even in older age groups (>70 years), the IFR varies from 1-5% depending on comorbidities and treatment access. As a basic principle, all-cause mortality (ACM) tends to increase with age. In the case of COVID-19, the presence of comorbid disease greatly modifies the influence of age on mortality [41]. For younger generations (<40 years), SARS-CoV-2 infection severity and fatality rates since 2020 have been comparable to those of influenza [42]. Even in countries that showed excess mortality in 2020, death rates among children were extremely low [43]. In Sweden, where 1.8 million children were allowed to freely attend school in 2020, zero COVID-19 deaths were recorded among them by summer 2021 [44].

Although randomized controlled trials are viewed as the gold standard for testing the safety and efficacy of medical products (due to minimizing bias), trials of limited scope can readily obscure the true safety and efficacy issues with respect to different segments of the population. In this case, the trials excluded key sub-groups, notably children, pregnant women, frail elderly persons, and immunocompromised individuals, as well as those with cancer, autoimmune disease, and other chronic inflammatory conditions [45]. Whereas the founding trials did not recruit individuals with comorbidities, vaccine recipients in the rollouts showed the actual presence of these underlying conditions. Rather than assess these well-known safety and comorbid risk concerns, the focus was narrowly placed on the potential for inflammatory lung injury as had been seen in COVID-19 patients and, many years earlier, in immunized animal models infected with SARS-CoV [46]. We are now beginning to recognize the folly of this narrow safety focus, as millions of severe and life-threatening events associated with the COVID-19 vaccines continue to be documented in the medical literature [47-51].

What did the pivotal trials reveal about overall (all-cause) mortality? After carefully analyzing the ACM for the Pfizer and Moderna trials, Benn and colleagues found 61 deaths total (31 in vaccine, 30 in placebo) and a mortality RR of 1.03 (0.63-1.71), comparing the vaccinated to placebo [52]. These findings can be interpreted as “no significant difference” or no gold-standard evidence showing these mRNA vaccines reduce mortality. The lack of significant differences in deaths between the study arms is noteworthy. The true mortality impact remains unknown in this context, and this fact alone is relevant, as it would be preferable to take a vaccine with good trial evidence of reduced mortality than to take a vaccine where trial evidence does not show convincing evidence of improved survival [53]. Similarly, a subsequent analysis of the Pfizer trial data concluded that mortality rates were comparable between vaccinated and placebo groups during the initial 20-week period of the randomized trial [54]. The fact that the mRNA vaccinations did not lead to a reduction in overall mortality implies that, if the injections were indeed averting deaths specifically attributable to COVID-19, any such reduction might be offset by an increase in mortality stemming from other causes, such as SAEs.

Even the six-month Pfizer trial failed to show any reduction in all-cause mortality [35]. Indeed, a reanalysis of the postmarketing data provided to the FDA suggests the opposite effect. The extended portion of the trial included four months of an unblinded period, in which most placebo participants crossed over to the vaccination group. During this phase, there were five additional deaths, including three in the original vaccine group and two among the placebo participants who chose vaccination [35]. When these five deaths are included as “vaccinated” deaths, the total count becomes 20 deaths in the vaccine group and 14 deaths in the placebo group, which would represent a 43% increase in deaths (not statistically significant due to small counts). In the FDA documents, however, a total of 38 deaths were reported, with 21 in the vaccine group and 17 in the placebo group, representing a 23.5% increase in all-cause deaths among those who received the two-dose primary series of BNT162b2 [55,56]. This suggests that the two placebo participants who died after mRNA vaccination were counted twice (i.e., both deaths were counted in each arm of the trial). To properly account for the five extra deaths, however, one should adjust the analysis based on person-months spent in each group. Applying this method, the total count was 36 deaths: 21 in the BNT162b2 arm and 16 in the placebo arm. Calculating the relative ACM risk, the vaccine group had a mortality rate of 0.105% (21 deaths out of 20,030), while the placebo group had a mortality rate of 0.0799% (16 deaths out of 20,030). The RR equation yielded a value of 1.3125 (95%CI 0.6851-2.5144, p=0.41), indicating a 31% higher ACM risk in the BNT162b2 group compared to the placebo group. The estimate may be considered conservative, as it does not assume that all placebo recipients chose to get vaccinated during the open-label phase of the trial.

For the Pfizer and Moderna registrational trials, Benn et al. also reported a non-significant 45% increase in cardiovascular deaths (RR=1.45; 95%CI 0.67-3.13) in the vaccine arms of the trials [52]. This outcome was consistent with numerous reports of COVID-19 vaccine-related cardiovascular pathology among both young and old segments of the population [57-63]. None of the mortality estimates from the trials are statistically significant. Nevertheless, the upward trends for both ACM and cardiovascular deaths are concerning. If the Pfizer trial had not been prematurely discontinued, and assuming death rates remain the same in both arms as observed in the first six months, the ACM difference would reach the standard threshold for statistical significance (p < 0.05) at approximately 2.8 years (34 months). The p-value is 0.065 at 2.5 years and 0.053 at 2.75 years (see Appendix 1). These calculations were independently confirmed by Masterjohn [64].

Absolute risk and the “number needed to vaccinate (NNV)”

One of the often-overlooked shortcomings of the registrational trials was the final reports’ exclusive focus on RR while omitting absolute risk reduction. The latter measure gives a better indication of a drug’s clinical utility than the former relative measure since it is scaled by the sample size [65]. RR is the ratio of COVID-19 symptom rates in the vaccine versus placebo groups, which was reported as 95% and 94.5% for the Pfizer and Moderna products, BNT162b2 and mRNA-1273, respectively [1,2]. Absolute risk refers to the probability of an outcome (in this case, symptoms of clinical infection), based on the number of people experiencing the outcome in relation to the population at large. It is typically calculated as the number of events that occurred in a study population divided by the number of people in that population. Both types of risk estimation are required to avoid reporting bias and to provide a more comprehensive perspective on vaccine efficacy [65]. Omitting the absolute risk statistics leads to overestimation of the clinical benefits of the vaccines [66]. In contrast with the 95% RR figure, the absolute risk reductions for BNT162b2 and mRNA-1273 were 0.7% and 1.1%, respectively [67]. These estimates were derived from publicly available data that ultimately enabled EUA for the vaccines to be granted by the FDA’s Vaccines and Related Biological Products Advisory Committee (VRBPAC) [68]. However, the data reviewed by the VRBPAC did not include absolute risk reduction measures, thus deviating from FDA’s guidelines, which state that both approaches are crucial in order to avoid the misguided use of pharmaceuticals [69]. Again, failing to provide the absolute risk and instead fixating only on RR generally results in an overestimation of vaccine benefits. Absolute risk statistics are also valuable when assessing and comparing safety measures such as AE rates.

An absolute risk reduction of approximately 1% for the COVID-19 mRNA vaccinations meant that a substantial number of individuals would need to be injected in order to prevent a single mild-to-moderate case of COVID-19. Specifically, the NNV to prevent one case of COVID-19 would be 142 (range 122-170) for the BNT162b2 injection and 88 (range 76-104) for the mRNA-1273 injection, respectively [65]. These numbers increase with age and depending on the variant [70]. The NNV is an interpretable and salient metric for assessing real-world impact, enabling us to gauge the potential benefits derived from vaccination. For any relatively healthy population (with minimal comorbidities), the risk-benefit profile with a high NNV could easily point to excessive harms.

It is imperative to carefully weigh all potential risks associated with the COVID-19 mRNA products. Should substantial harms be linked to their use, the perceived “reward” conveyed by the NNV would necessitate a re-appraisal. For example, assuming an NNV of 119 and an IFR of 0.23% (both conservative estimates), approximately 52,000 vaccinations would be needed to prevent one COVID-19-related death. Thus, for the BNT162b2 injection, a generous estimate would be two lives saved from COVID-19 for every 100,000 courses of the biological. Given the evidence of trial misconduct and data integrity problems (see next section), we conjecture that this estimate is an “upper bound”, and therefore the true benefit is likely to be much lower. Regarding potential harms, assuming 30% false-positive reports and a moderate under-reporting factor of 21, we calculate a risk of 27 deaths per 100,000 doses of BNT162b2. Thus, applying these reasonable, conservative assumptions, the estimated harms of the COVID-19 mRNA vaccines greatly outweigh the rewards: for every life saved, there were nearly 14 times more deaths caused by the modified mRNA injections (for details, see Appendix 2).

Underreporting of harms and data integrity issues

Underreporting of severe harms, including SAEs, is another important concern that often garners scant attention in the public domain. Notably, severe harms that significantly impede daily activities and quality of life are universally underreported in randomized trials, particularly in industry-sponsored studies [71]. Such AEs may be most common in mRNA-vaccinated individuals who are subsequently infected with SARS-CoV-2. While, in principle, systematic reviews of randomized trials serve as a reliable source of evidence, the reporting of serious harms is invariably missing from the drug trial reports [72]. This dearth of reporting seems exceptionally evident in the context of vaccine trials [73-75]. In the case of the COVID-19 vaccine trials, the underreporting was also situational, as participants were unblinded in the open-label phase of the Pfizer trial, and placebo recipients were offered the vaccine within only a few weeks of the EUA. The early unblinding occurred without allowing sufficient time to identify late-occurring or diagnosed harms associated with the vaccines [15]. Was this necessary, given that none of the deaths in the Pfizer trial were attributed to COVID-19 as the primary cause, and given the very low IFR for a relatively healthy population [40]?

Classen notes that the trial coordinators employed a haphazard approach to AE monitoring and thus the potential harmful impact of these biologicals on health outcomes was more substantial than is usually acknowledged [49]. Investigators prioritized the documentation of COVID-19 events while prospectively tracking patients for “solicited” AEs for a duration of approximately seven days post immunization. “Unsolicited” AEs were subsequently reported for a period of 30-60 days. Among the trial participants were individuals with limited education and elderly individuals (possibly with cognitive impairment) [49]. The ability of such individuals to competently recognize and report serious AEs is questionable. Moreover, the original trial reports did not include data on serious non-infectious events, including fatalities, that occurred beyond the 30-60-day reporting period [49]. By contrast, COVID-19 infections were continuously monitored from the time of immunization (a form of information bias). Both Pfizer and Janssen showed leniency in recording AEs, restricting the documentation of “solicited” events to a safety cohort representing less than 20% of the overall study population. These findings align with prior studies showing that only a small proportion, generally 5%, of AEs are typically reported in pharmaceutical company-sponsored trials [76].

To make matters worse, the public was never allowed access to the registrational trials’ raw data, thus precluding independent verification of AEs by the scientific community (these were revealed later on, after widespread distribution of the inoculations) [77]. Such secrecy may have enabled the industry to more easily present an inflated and distorted estimate of the genetic injections’ benefits, along with a gross underestimation of potential harms.

A recent forensic analysis of Pfizer’s six-month trial data revealed that many deaths in the trial occurred after the cutoff date used to create the briefing booklet reviewed by the FDA and resulting in the authorization of the vaccine; this effectively concealed mortality data from the decision-making part of the EUA process [54]. Pfizer’s original application for the EUA described the trial results only up to the data cutoff date of November 14, 2020. However, deaths and other SAEs continued to occur afterward, even before the definitive VRBPAC meeting to authorize the mRNA vaccine. During the initial 33 weeks of Pfizer-BioNTech Clinical Trial CA4591001, which spanned 153 clinical trial sites in more than seven different countries, a total of 38 subjects passed away. The 38 trial subjects were listed in the Pfizer-BioNTech six-month Interim Report [35]. These events occurred in chronological order within the 33-week period commencing on July 27, 2020, and concluding on March 13, 2021. To visually represent this data, Michels et al. created a bar graph illustrating the number of subject deaths per week (Figure 1). The number of subject deaths in both the BNT162b2 (“vaccinated”) and placebo arms of the trial is depicted separately. The graph also includes a plot illustrating the cumulative number of deaths in each arm, measured at the end of each week. Solid bars represent subjects who received the BNT162b2 injection, while gray bars represent those who received a placebo, and hatched bars represent subjects who initially received a placebo but were unblinded and subsequently administered BNT162b2. Additionally, the authors included a linear graph that displays the cumulative number of deaths in each trial arm. A solid line corresponds to BNT162b2-injected subjects, while a dotted line represents the placebo group [54].

**Figure 1:** Analysis of Pfizer trial’s weekly mortality over a 33-week period This representation of the Pfizer trial by Michels et al. [54] showcases the weekly count of subject deaths from July 27, 2020, to March 13, 2021. Solid bars denote BNT162b2 recipients, gray bars signify the placebo group, and hatched bars represent previously unblinded placebo subjects who later received BNT162b2. The solid line represents the cumulative death count for the BNT162b2 group and the dotted line for the placebo group. Image Source: Michels et al., 2023 [54]; Published with permission by authors under CC BY-NC-ND 4.0 Deed (Attribution-NonCommercial-NoDerivs 4.0 International)

Notably, the unblinded placebo recipients who later received BNT162b2 are combined with the BNT162b2 “vaccine group” for this analysis [54]. To provide context, the registrational trial can be divided into three distinct periods. The first is the “Blinded placebo-controlled period,” which spanned from July 27, 2020, to December 10, 2020. The second phase is the “Open-label follow-up period,” encompassing the timeframe from December 11, 2020, to January 24, 2021. The final period is the “Open-label observation period,” which extended from January 25, 2021, to May 13, 2021 [35,78]. The initial placebo subject death was recorded in Week 5, while the first death among BNT162b2 subjects occurred in Week 7.

The first 12 weeks of the trial saw very few deaths, likely due to ongoing enrollment of new subjects. The plots illustrating the cumulative number of deaths in both arms appear to closely align until around Week 20, after which they diverge (Figure 1). Beyond Week 20, the rate of deaths in the placebo arm decreased and eventually stabilized by Week 30. In contrast, the number of deaths among BNT162b2 subjects continued to rise at a consistent rate. This reduced rate in the placebo arm was likely a result of the diminishing number of unvaccinated placebo subjects remaining in the trial, stemming from the unblinding and vaccination process initiated after December 11. Despite the low overall death count, it is likely that the general public’s perception of the vaccines would have been far less favorable had they known that the mortality rate had continued to increase among the mRNA-vaccinated participants [54]. The data for Figure 1 by Michels et al. [54] were obtained directly from Pfizer’s Six-Month Interim Report [35]. Moreover, Michels et al. [54] compared the reported number of deaths to an age-stratified estimated number based on US data from 2019 [79]** **and determined that Pfizer’s reported number of 38 deaths is about 17% of what would be expected for the US population.

Alarmingly, drawing from Pfizer’s Six-Month Interim Report, Michels and colleagues found evidence of a substantial increase in the number of deaths due to cardiovascular events in BNT162b2 vaccinated subjects that the vaccine manufacturer did not report [54].For their published peer-reviewed analysis, the researchers were able to access the narrative reports on a few critical subjects that provided explicit notification of the subject’s date of death prior to November 14, 2020 [54]. Protocol C4591001 required immediate reporting of SAEs, including death or hospitalization, within a 24-hour window, a guideline likely followed by the trial site staff. Nevertheless, Pfizer used the dates that the death was recorded in the subject’s Case Report Forms, which Pfizer maintained. The Michels et al. investigation uncovered a consistent pattern of reporting delays of the date of death on subjects’ Case Report Forms across the entire trial [54]. These delays were greatest in vaccinated subjects who died prior to November 14, 2020. If Pfizer had used the actual death dates in their EUA application, two additional vaccinated subjects would have been included in the EUA application. This discrepancy was crucial, as all vaccinated subject deaths (four of four) and half the placebo deaths (two of four) were cardiac-related. The forensic analysis revealed that 75% of the deaths in vaccinated subjects and 33.3% of those in the placebo group were cardiac-related [54]. Among the 14 subjects experiencing cardiac SAEs, 11 were individuals who received the BNT162b2 vaccine, and three were from the Placebo-only trial arm, a 3.7-fold increase (OR 3.7, 95%CI 1.02-13.2, p = 0.03) [54]. It is noteworthy that neither the original trial paper by Thomas et al. nor Pfizer’s Summary Clinical Safety report acknowledged or commented on this crucial safety signal [35,78].

In hindsight, the previously undisclosed observation that twice as many cardiac deaths occurred proportionately among vaccinated compared to unvaccinated subjects in the Pfizer trial would likely have prompted the FDA’s reevaluation, especially considering the later accumulated data by December 10, 2020, where 17 deaths had occurred [54]. Delays in documenting these patients’ fatalities in their Case Report File, coupled with the omission of the actual date of death, effectively concealed their deaths during the crucial phase of the EUA approval process, masking the cardiac SAE signal [54]. In short, the various reporting delays and omissions, if they had been openly discussed and considered by the VRBPAC, might have prolonged the authorization process. The improper reporting and insufficient scrutiny by the VRBPAC may have ultimately enabled Pfizer to manipulate the trial results and obscure the cardiac death signal. Recent in vivo animal studies demonstrate that “in isolated cardiomyocytes, both mRNA-1273 and BNT162b2 induce specific dysfunctions that correlate pathophysiologically to cardiomyopathy” [80]. In principle, then, cardiomyocytes cannot be excluded from the biodistribution of the LNP-mRNA, and every new mRNA product has the potential to cause life-threatening heart problems, including cardiomyopathy and cardiac arrest.

Beyond these omissions in SAE reporting, the official reporting of trial results was also problematic. The trial data Pfizer submitted for the EUA application revealed a puzzling trend when comparing COVID-19 incidence between the mRNA-injected and placebo groups: a striking divergence after day 12 following the first BNT162b2 dose [81,82]. While the placebo group continued to see new cases, the BNT162b2 group’s infection rate abruptly halted, suggesting sudden, uniform immunity onset at day 12. Such an abrupt and complete response on day 12 contradicts biological plausibility, given that such immunological responses would realistically tend to register in a more gradual way in a group context. Moreover, Pfizer failed to provide the data for individuals receiving only one dose. Figure 2 from the same trial report [83], adapted by Palmer et al. [82], showing neutralizing antibody titers on the day of the first injection (D1) and various subsequent days, depicts the gradual rise of neutralizing antibodies to SARS-CoV-2 following the mRNA inoculation. This contradicts the notion of rapid, full clinical immunity. By day 21, after the first dose, neutralizing antibodies only slightly increased, peaking on day 28, well after most individuals would have received their second dose. This inconsistency between clinical and antibody data raises doubts about the graphic depiction of sudden immunity on day 12, casting suspicion on its validity. Figure 2 shows two charts sourced from the European Medicines Agency (EMA) assessment report on Pfizer's trial data [83].

**Figure 2:** Charts illustrating Pfizer trial irregularities in reporting of COVID-19 cases and humoral immune responses (antibody titers) This  indicates an unusual pattern post day 12 following the BNT162b2 injection. While the placebo group continued experiencing cases, the BNT162b2 group showed a sudden decline in infection rates, suggesting unexpected immediate immunity. Image source: Palmer M, et al., 2023 [82];  Reproduced under Creative Commons Attribution-NonCommercial-ShareAlike 4.0 International License (CC BY-NC-SA 4.0). Data was extracted from the European Medicines Agency (EMA) report, referencing Figures 9 (A) and 7 (B) [83].

When Pfizer’s Six-Month Interim Report of Adverse Events (C4591001) revealed a total death count of 38 [35], the number seemed unexpectedly low for a clinical trial involving 44,060 participants amidst a pandemic. To investigate, Michels and colleagues estimated the anticipated deaths based on US mortality rates in 2020, presuming comparability across participating countries [54]. With 132 trial sites in the US and 80% of subjects, they estimated that 222 deaths should have occurred between July 27, 2020, and March 13, 2021, making the observed 38 deaths only 17% of the projected number. Most of the trial sites had fewer deaths than anticipated, possibly attributed to a considerable percentage of “Lost to Follow-up” subjects (4.2% of randomized subjects), including 395 unique subjects within the study period. While some sites recorded negligible losses, others exhibited substantial figures, up to 5% of the site’s subjects [54]. These numbers likely contributed to the seemingly low overall death count and should have prompted increased efforts to locate these individuals. Losing track of nearly 400 study participants in the follow-up observation period could have substantially compromised the validity and generalizability of the results. The missing data can produce biased estimates, leading to invalid conclusions. This could result in a distortion of vaccine efficacy and underestimation of SAEs (including deaths), thus misrepresenting the safety profile of the mRNA products. In short, Pfizer’s failure to minimize participant attrition seriously undermined the accuracy and reliability of the six-month study’s conclusions.

According to a retrospective analysis by Gulbrandsen and colleagues, the Pfizer trial data showed a significant association between the mortality rate and time since the injection in both the vaccine and placebo arms [84]. A minimal number of deaths were recorded during the initial 80 days, but a significant mortality increase was observed around the 100-day mark post-injection, indicating a pattern that cannot be attributed to chance. Remarkably irregular trends are also evident in the cardiac SAEs within the trial. Nearly half of all the cardiac events manifested within the initial 50 days following the injection, despite the constant risk exposure anticipated for the first 140 days. Oddly, a dramatic surge in cardiac SAEs was observed around the 100-day mark from the first injection in both the placebo and vaccine groups, coinciding with the heightened death rate. Examining the predominant medical diagnoses before participation in the trial revealed yet another aberrant trend: all nine of the most prevalent pre-existing diagnoses were more commonly found among participants in the placebo arm. Moreover, there was a notable contrast in the ages of deceased participants between the two groups. These observed patterns were unlikely to occur randomly. The only plausible explanation that aligned with these anomalous trends was that the SAE records among vaccine recipients were altered, relocating them to the placebo arm post occurrence [84].

These concerns are further compounded by revelations concerning substandard research practices and inadequate data management in the pivotal trials. A whistleblower report by a former employee of the contract research organization responsible for enrolling patients in Pfizer’s pivotal trial raises significant questions regarding data integrity and the safety of trial participants [85]. Among the trial conduct issues documented were failure to report protocol deviations, improper storage of vaccines, mislabeling of laboratory specimens, and lack of timely follow-up for patients experiencing AEs, possibly leading to underreporting. In terms of regulatory oversight, the FDA inspected only nine out of the 153 study sites involved in the Pfizer trial [86].

Finally, an unblinding of participants occurred early in the trial, potentially on a wide scale across different study sites. Participants were not presented with clear information regarding potential AEs in both trial protocols and consent forms [87]. Some parts of the consent form were misleading and merely intended to elicit participation that might not otherwise have occurred if the volunteers had been made aware that what was promised in theory or “on paper” was unlikely to happen in reality [87]. As a result, participants were not being granted truly informed consent; the potential injuries and AEs most likely to be caused by the vaccinations were never openly stated.

This lack of informed consent carried over into the real-world setting following the EUA. For example, not publicly disclosing the Pfizer trial’s exclusion of pregnant women is arguably among the CDC’s most egregious oversights when asserting the safety of COVID-19 vaccine administration during pregnancy [1]. The Nuremberg Code established patients’ rights to voluntary informed consent in the aftermath of World War II [88]. US courts consistently support informed consent as a fundamental right for patients’ autonomy [89]. Informed consent procedures must provide clear distinctions between risks that are frequently observed, risks that occur rarely, and the more obvious risk of lack of effectiveness or waning immunity, which is separate from the risk of SAEs. Whether in a clinical trial or free-living real-world setting, informed consent is essential to providing a clear understanding of the potential risks associated with receiving a genetic vaccine. Throughout the pandemic, healthcare workers were duty-bound to provide clear risk-benefit information to patients. In practice, however, informed consent was non-existent, as information sheets were blank [90], and vaccinees were never informed of potential risks beforehand.

Shifting narratives, illusions of protection

The ability to halt or greatly limit infection is generally considered essential to vaccine effectiveness. Nevertheless, the registrational trials by Pfizer and Moderna were not designed to address this issue. The endpoint of the trials was the reduction of symptoms associated with COVID-19 [1,2], even though the public was subsequently told by the CDC that the COVID-19 products would stop transmission [91]. Moreover, asymptomatic transmission was shown to be extremely minuscule [92]. Since 2021, the scientific community has known that the COVID-19 mRNA products do not prevent either transmission or infection [93]. Even experts sponsored by the vaccine industry admitted to a maximum reduction in transmission of 61% in 2021 [94]. The Omicron subvariants are associated with a 30-50% reduction in transmission following administration of the boosters [95-97]. The benefit is incremental and transient, with protection against Omicron infection lasting only a few months [93]. Even though antibody titers against SARS-CoV-2 are higher following the injection, these levels decline faster in the mRNA recipients compared to individuals with natural infection [98]. The impact of reduced disease severity among COVID-19-vaccinated individuals on the risk of causing secondary infections has never been systematically investigated in controlled clinical trials [93].

The best evidence for the failure of the COVID-19 mRNA vaccine’s ability to confer protection against COVID-19 comes from two large cohort studies of employees within the Cleveland Clinic Health System (CCHS) after the bivalent mRNA boosters became available [99,100]. In the first study (n=51,017), COVID-19 occurred in 4,424 (8.7%) during the 26-week observation period [99]. In terms of preventing infections by the three prevailing Omicron subvariants, the vaccine effectiveness was 29%, 20%, and a non-significant 4%, respectively [99]. No protection was provided when the XBB lineages were dominant. Notably, the risk of “breakthrough” infection was significantly higher among those who received the earlier vaccine, and a higher frequency of vaccinations resulted in a greater risk of COVID-19 [100]. In a second CCHS cohort study (n= 48,344), adults who were “not up-to-date” by the CDC definition had a 23% lower incidence of COVID-19 than those “up-to-date” with their vaccinations [100]. These findings are further reinforced by multiple real-world studies showing rapidly waning protection against Omicron infection after the boosters [101]. The vaccine effectiveness against laboratory-confirmed Omicron infection and symptomatic disease rapidly wanes within three months of the primary vaccination cycle and booster dose [97].

Figures 3-4 present the surprising findings from these two Cleveland Clinic studies. Figure 3 displays the earlier study's findings, with a cumulative incidence of COVID-19 for study participants stratified by the number of mRNA vaccine doses previously received. Day 0 was September 12, 2022, the date the bivalent vaccine was first offered to CCHS employees. Case rates were clearly increasing in tandem with greater frequency of mRNA injections [99]. Figure 4 presents another unexpected finding, this time from the second Cleveland Clinic study, with a Simon-Makuch hazard plot comparing the cumulative COVID-19 incidence in the “up-to-date” and “not up-to-date” with respect to CDC-defined vaccination status. Day zero was January 29, 2023, the day the XBB lineages of the Omicron variant became dominant in Ohio. For both charts, point estimates and 95%CIs are shown along the x-axis [100].

**Figure 3:** Cleveland Clinic study showing increasing COVID-19 cases with increasing mRNA vaccinations Cleveland Clinic study demonstrating COVID-19 incidence among participants based on the number of prior mRNA vaccine doses received. The study shows rising case rates associated with increased COVID-19 mRNA vaccine doses. Image Source: Shrestha et al., 2023 [99]; Open Access article with public sector information, licensed under the Open Government Licence v3.0 (http://www.nationalarchives.gov.uk/doc/open- government-licence/version/3/)

**Figure 4:** Cleveland Clinic study showing increased COVID-19 cases for subjects most "up to date" with mRNA vaccinations Cleveland Clinic study comparing cumulative COVID-19 incidence between "up-to-date" and "not up-to-date" individuals based on CDC-defined vaccination status. The plot includes point estimates and 95% confidence intervals along the x-axis. Image Credit: Shrestha et al., 2023 [100]; Open access, licensed under CC BY 4.0 Deed (Attribution 4.0 International)

With the product efficacy profile now firmly in question, the vaccine enterprise has embraced two narratives to justify the ongoing use of COVID-19 vaccinations. The first is that while the COVID-19 mRNA products may not block infections, these products still protect against severe disease, hospitalization, and mortality. The second narrative states that the protection associated with the mRNA inoculation, when combined with natural infection, is superior to natural infection (and thus natural immunity) alone.

The first narrative posits a counterintuitive dichotomy between the two forms of protection, protection against infection versus protection against severe disease, and seems to imply their independence. As an encapsulation of this dichotomy, a 2022 Israeli study report states that the “protection against confirmed infection appeared short-lived, whereas protection against severe illness did not wane during the study period" [102]. However, is it reasonable to contend that protection against severe illness and mortality remains intact even after the rapid decline in protection against infections? To address this issue, Ophir and colleagues conducted a meticulous analysis of prominent data from clinical trials, large observational studies from Israel, and contemporary dashboards of statistics [103]. The authors noted “multiple methodological and representational constraints, including short, and sometimes arbitrary or uneven follow-up periods, uneven exclusion criteria and COVID-19 testing levels, selection biases, and selective reporting of results. But most importantly, the documented, conditional probability of death and severe illness (i.e., the percentage of severe illness and death cases among those infected with the virus) did not differ between the treatment and the control groups of the various clinical and observational efficacy studies" [103]. The authors concluded that there was no valid evidence to substantiate the claim that getting a second COVID-19 mRNA booster effectively prevents severe illness and mortality [103].

The second alternative narrative focuses on the phenomenon of hybrid immunity, the combined protection obtained from natural infection followed by the booster. In those individuals recently exposed to SARS-CoV-2 infections, COVID-19 vaccine-induced immunity is believed to surpass natural immunity because it generates a more robust antibody response and broadens the spectrum of antibodies generated [104]. These robust, broad-based humoral responses entail the production of memory B cells at levels 5-10 times higher than those achieved through either infection or vaccination alone [105]. By now, most if not all individuals in developed countries have been infected by SARS-CoV-2. Once informed of the additional protection afforded by hybrid immunity, laypersons cognizant of having a history of infection may be more inclined to embrace ongoing boosters. Nonetheless, given the relatively low severity of Omicron, is the additional antibody production truly necessary? One also needs to consider the potential risks of this increased antibody production. Because the Omicron subvariants are constantly mutating, many of the antibodies generated by current vaccines are non-neutralizing. The potential overproduction of non-neutralizing antibodies could lead to the phenomenon of vaccine-associated enhanced disease (VAED), which is based in part on antibody-dependent enhancement [106]. To date, there have been only a few reports of mild VAED in COVID-19 vaccination in animal models and no documented cases in humans [107]. With repeated boosters, however, VAED could eventually impact the long-term safety of the mRNA vaccinations.

In the context of hybrid immunity, the most serious immunological pitfall pertains to SARS-CoV-2 infection occurring after the COVID-19 mRNA injection, when S-protein production is already systemically increased. It was originally assumed that prior vaccination might lessen the severity of the infection and reduce the risk of severe COVID-19 illness. In the post-vaccination period, the immune system would be primed for responding more robustly to a subsequent infection within a few weeks after completing the full series. However, the opposite scenario can also unfold due to the circumvention of innate immune responses, together with the above-mentioned overproduction of non-neutralizing antibodies and inadequate protection against severe disease [108]. COVID-19 vaccinations are known to cause innate immune suppression via profound impairment in type I interferon signaling along with disruption of regulatory control of protein synthesis and cancer surveillance [26]. Excessive production of non-neutralizing antibodies could increase the risk of autoimmune reactions by cross-reacting with host tissues instead of the virus, thereby triggering inflammatory autoimmune reactions via molecular mimicry [109-111]. These mechanisms may collectively raise the risk of autoimmune inflammatory pathologies, including cancers, cardiovascular diseases, and many other diseases with a chronic inflammatory etiology [112,113]. (For a discussion of the mechanistic basis for adverse events, please see the section, “Mechanisms underlying AEs”.)

Up to this point, when considering the SAEs, we have focused primarily on those effects associated with Pfizer’s mRNA product, BNT162b2, drawing from the six-month trial data as well as the 393-page confidential document released on August 2022, revealing close to 1.6 million AEs [114]. In the context of hybrid immunity, it is important to note that the Moderna product, mRNA-1273, generates a substantially stronger immune response, resulting in lower rates of symptomatic infection and severe COVID-19 outcomes when compared to BNT162b2 [115]. Those who fixate on these infection-preventing benefits, however, may tend to overlook the potential harms: mRNA-1273 has exhibited significantly higher risks of SAEs compared to BNT162b2, according to clinical trials, survey-based studies, and a government-sponsored surveillance study [1,2,116-120]. This shows the unsavory trade-off between increased protection against Omicron infection on the one hand and a substantial risk of vaccine-induced SAEs on the other.

In a recent study of nearly five million adults, those who had a SARS-CoV-2 infection within 21 days post injection showed an eight-fold increased risk of ischemic stroke (OR=8.00, 95%CI 4.18-15.31) and a five-fold increased risk of hemorrhagic stroke when compared to vaccinees without concurrent infection (OR=5.23, 95%CI 1.11-24.64) [121]. The risk was highest for those receiving the mRNA-1273 injections. Thus, SARS-CoV-2 infection close to the time of vaccination produced a strong association with early incidence of ischemic and hemorrhagic strokes [121]. Again, with a hybrid immunity approach, the potential harms may greatly outweigh the rewards.

Natural immunity carries none of these risks and is more than sufficient against the mild virulence of Omicron subvariants. Much evidence now indicates that natural immunity confers robust, durable, and high-level protection against COVID-19 severe illness [122-126]. A large United Kingdom (UK) study of over 30,000 healthcare workers, having a prior history of SARS-CoV-2 infection, showed an 84% reduced risk of reinfection, with a median protective period of seven months [125]. In a large observational study in Israel, previously infected individuals who remained unvaccinated were 6-13 times less likely to contract the virus compared to those who were vaccinated [122]. Among 32,000 individuals within the same healthcare system, vaccinated individuals had a 27-time higher risk of developing symptomatic COVID-19 and an eight-time higher risk of hospitalization compared to their unvaccinated counterparts [122].

After recovering from COVID-19, the body harbors long-lived memory immune cells, indicating an enduring capacity to respond to new infections, potentially lasting many years [127]. Mounting evidence suggests that the training of antibodies and induction of T-cell memory resulting from repeated natural infection with Omicron can augment the mitigation of future infections [128,129]. In a recent cohort study, children who had experienced prior infection showed long-lasting protection against reinfection with SARS-CoV-2 for a minimum of 18 months [130]. Such children between the ages of five and 11 years demonstrated no decline in protection during the entire study, while those aged 12-18 experienced a mild yet measurable decline in protection over time [130]. For these younger generations in particular, natural immunity is more than sufficient and of course vastly safer than the mRNA inoculations.

Analyses of serious harms to humans

We now review what is known about the AEs and SAEs reported in the registrational trials, including data that regulatory agencies and drug safety surveillance studies revealed following the EUA. As early as 2014, Sahin and colleagues had warned of the potential dangers of the mRNA vaccine technology, specifically cautioning that the encoded antigen should be investigated for multiple disease risks [131]. Surveys show that the primary concern expressed by parents regarding their children receiving the COVID-19 vaccines is not vaccine effectiveness but rather the potential AEs [132,133]. In a survey of US parents, concerns about the unprecedented speed of the mRNA vaccines’ development (and, by implication, the rapid authorization process) were ranked just above concerns about harmful side effects [133]. The risks may vary depending on the number and frequency of COVID-19 vaccine doses. Whereas some authors have observed fewer AEs after the second dose [134], others have reported an increased incidence [116]. Sultana et al. reported varying trends in AEs after the second dose for both mRNA products, albeit with a higher frequency of AEs following the second-dose administration of the Moderna vaccine [135].

The most compelling revelations regarding the adverse impacts of these products have come from a comprehensive re-analysis of the trial data, with a primary focus on the more serious outcomes, including fatalities. Applying rigorous methodology, Fraiman and colleagues conducted an in-depth investigation and analyzed the interim datasets for the Pfizer and Moderna trials, encompassing approximately four months of observation following the commencement of the trials [50]. SAEs were defined as events that led to any of the following outcomes: death, life-threatening conditions, inpatient hospitalization or extension of existing hospitalization, persistent or significant disability/incapacity, a congenital anomaly/birth defect, or a medically significant event based on medical judgment. The risk of vaccine-related SAEs was divided into general SAEs and AEs of special interest (AESIs), as identified by the Brighton Collaboration criteria adopted by the World Health Organization [136].

For both the Pfizer and Moderna trials combined, there were about 125 SAEs per 100,000 vaccine recipients, which translates into one SAE for every 800 vaccinees [50]. Because the trials avoided the most frail as participants, one would expect to see even higher proportions of SAEs in the population-wide rollouts. Remarkably, the Pfizer trial exhibited a 36% higher risk of SAEs in the vaccine group compared to the placebo, with a risk difference of 18.0 (95%CI 1.2-34.9) per 10,000 vaccinated; risk ratio 1.36 (95%CI 1.02-1.83). These findings stand in sharp contrast with the FDA’s initial claim that SAEs reported by the two pivotal trials were “balanced between treatment groups” [15,50]. The discrepancy may be partly explained by the fact that the FDA was focusing only on individual participant data, and yet many of those individuals were experiencing multiple SAEs. Instead of analyzing individuals, Fraiman et al. focused on total SAEs to take into account the multiple, concurrent events [50]. When the SAEs were viewed collectively, the risks in the vaccine group were substantially elevated beyond those previously determined by the FDA.

For their risk-benefit assessment, Fraiman’s team considered the excess risk of serious AESIs in the vaccine group versus the risk of COVID-19 hospitalization in the placebo group [50]. This analysis was based on published reports from the vaccine companies’ sponsors and FDA presentations. Remarkably, according to Fraiman et al., the Pfizer trial exhibited a four-fold higher risk of serious AESIs compared to the risk of COVID-19 hospitalizations (10.1 AESIs vs. 2.3 hospitalizations per 10,000 participants, respectively), while the Moderna trial demonstrated a more than two-fold higher risk (15.1 AESIs vs. 6.4 hospitalizations per 10,000 participants, respectively) [50]. These findings indicate a much stronger degree of vaccine-related harm than initially estimated during the time of EUA. To put these findings in perspective, the official SAE rate for other vaccines is only 1-2 per million [137]. Fraiman et al.’s estimate based on the Pfizer trial data (1,250 SAEs per million) exceeds this benchmark by at least 600-fold.

Analyses of two large drug safety reporting systems in the US and Europe revealed over 7.8 million AEs reported by approximately 1.6 million individuals following COVID-19 vaccination [47]. When compared to individuals aged 18-64 years, the older age groups exhibited a higher frequency of death, hospitalizations, and life-threatening reactions, with RR estimates ranging from 1.49 (99%CI 1.44-1.55) to 8.61 (99%CI 8.02-9.23). Signals were identified for myocardial infarction, pulmonary embolism, cardio-respiratory arrest, cerebral infarction, and cerebral hemorrhage associated with both mRNA vaccines. These signals, along with ischemic strokes, were confirmed by a large disproportionality analysis [48]. In an independent risk-benefit analysis, BNT162b2 produced 25 times more SAEs than the number of severe COVID-19 cases prevented [51]. Such an uneven risk-benefit calculus reinforces the findings from the Skidmore survey, which estimated that the total number of US fatalities due to COVID-19 mRNA vaccinations in 2021 alone was 289,789 (95%CI 229,319-344,319) [138]. A physician and survey research specialist helped to validate the survey, and the sample (obtained by Dynata, the world’s largest first-party data platform, based in Connecticut, US) was deemed representative of the US population [138].

Finally, autopsy studies have provided additional evidence of serious harms. In a comprehensive systematic review with full independent adjudication, 74% of autopsy findings (240 out of 325 cases), were judged to have been caused by the COVID-19 mRNA products [139]. The mean time from injection to death was 14.3 days, and the vast majority of deaths had the cardiovascular system as the single fatal organ system injury to the body. These findings are reinforced by those of a more recent adjudicated autopsy review of mRNA vaccine-induced myocarditis (28 deaths, all of which were attributed to the injections) [140] as well as a previous autopsy study of mRNA vaccine recipients that did not have the advantage of independent adjudication [141]. Based on multiple autopsy studies, German pathologists led by the late Arne Burkhardt have documented the presence of vaccine-mRNA-produced S-proteins in blood vessel walls and brain tissues through immunohistopathological-staining [142,143]. These findings help explain the wide range of well-documented COVID-19 vaccine-induced toxicities that impact the nervous, gastrointestinal, hepatic, renal, hematological, immune, and reproductive systems [25,144,145]. Post-mortem examinations are critical for identifying potential SAEs of the mRNA inoculations. However, as clinics and hospital administrations have a large vested interest in the COVID-19 vaccines’ distribution, the common administrative practice of discouraging autopsies and postponing autopsy reports only serves to undermine comprehensive risk assessment, perpetuate public misconceptions regarding safety, and weaken public health policymaking [145].

Quality control issues and process-related impurities

Given the novelty of the mRNA technology used in the SARS-CoV-2 vaccines, it would be prudent to establish regular production inspection and quality assurance along with long-term safety monitoring protocols and to perform the requisite tumorigenicity, genotoxicity, neurotoxicity, immunotoxicity, and reproductive toxicity studies. The fact that no safety and toxicity studies appropriate for these gene-based or GTP products were ever performed is concerning.

A key issue that could help explain why some individuals succumb while others do not is vaccine type and batch variability. Due to the inherent instability of mRNA technology, some batches may contain extremely low levels of intact mRNA [146]. Some batches were contaminated with double-stranded RNA (dsRNA), as documented by the EMA for both the Pfizer and Moderna products [147,148]. The dsRNA has a high potential to trigger immune-inflammatory reactions such as myocarditis [149].

Quality control is central to any discussion of batch variability and process-related impurities, and yet, in practical terms, evaluating such control for individual vials is not feasible. In a paper published in 2021, Yu et al. hypothesized that variability in adverse reactions might be caused by quality differences among different batches or even different individual vials, due to variabilities in both contaminants and handling histories [150]. The requirement of maintenance at extremely low temperatures may not always be practical, and the consequences of improper handling (e.g., cold chain breaching) are not well characterized.

The issue of batch variability is further complicated by recent findings of DNA contamination in the mRNA vaccines [151]. In an analysis of multiple vials of the bivalent Pfizer and Moderna mRNA products, McKernan et al. found “high levels of DNA contamination in both the monovalent and bivalent vaccines” that were “orders of magnitude higher than the EMA's limit” of 330 nanograms of DNA per milligram of RNA [152]. The DNA process-related impurities also exceeded the safety limits of the FDA (10ng/dose).

In a follow-up attempt to disprove this claim, Buckhaults and his genomics research team examined two batches of Pfizer mRNA vials and confirmed contamination with the plasmid DNA vector that had been used as the template for mRNA vaccine production [8,153]. At a South Carolina Senate hearing, Buckhaults reported having consistently sequenced substantial quantities of plasmid DNA, 200 billion DNA fragments per vial [153].

A surprising and potentially alarming discovery was the presence of the Simian virus 40 (SV40) promoter in samples of the Pfizer vaccine, which was notably absent from the Moderna vaccine samples [151]. In October 2023, the regulatory agency Health Canada confirmed the presence of this genetic sequence in mRNA vaccine samples [154]. SV40, an oncogenic DNA virus originally isolated in 1960 from contaminated polio vaccines, induces lymphomas, brain tumors, and other malignancies in laboratory animals [155]. Immunological data from cancer patients have indicated that their sera had a higher prevalence of antibodies against SV40 compared to healthy subjects [156]. A meta-analysis based on pooling diverse data from 1,793 cancer patients identified a significant excess risk of SV40 in association with brain tumors, bone cancers, non-Hodgkin’s lymphoma, and malignant mesothelioma [157]. It seems improbable, however, that SV40 exposure alone results in human malignancy, as suggested by the absence of a cancer epidemic following the distribution of SV40-contaminated polio vaccines. A more likely scenario is that SV40 functions as a cofactor in the genesis and progression of tumors, as indicated by laboratory studies revealing its cocarcinogenic potential with asbestos, an established carcinogen [158].

The SV40 promoter has found potential use as an enhancer in gene therapy treatments based on DNA plasmids. In a 2001 study on somatic gene delivery to skeletal muscle cells, it was shown that incorporation of the SV40 enhancer into DNA plasmids could increase the level of exogenous gene expression by a factor of 20 [159]. According to an insightful editorial on the implications of process-related impurities, the packaging of DNA fragments into lipid particles enhances the possibility that the DNA fragments will integrate into the human genome [160].

While absent in the vials utilized during the registrational trials, the SV40 promoter has been identified in all tested BioNTech vials drawn from batches that have been distributed to the public. On December 6, 2023, Florida’s surgeon general Joseph Ladapo contacted the FDA and CDC with questions about safety assessments and the discovery of billions of DNA fragments per dose of the mRNA vaccine products [161,162]. A week later, the FDA responded in writing by citing genotoxicity studies (which are inadequate for evaluating the risk of DNA integration) and by blurring the distinction between the SV40 promoter/enhancer and SV40 proteins, erroneously treating these elements as interchangeable [162]. Because the agency has thus far failed to provide any evidence of conducting DNA integration assessments to address the risks highlighted by the agency itself back in 2007, Ladapo called for a complete halt on the use of all COVID-19 mRNA vaccines [161,162]. In a Brownstone Institute article, mRNA vaccine developer Robert Malone strongly criticized the FDA’s unwillingness to evaluate the potential risks of the contaminant DNA [163].

A joint statement offered by an international expert advisory panel sponsored by the World Council for Health included the following: “There are multiple completely undeclared genetic sequences in both Moderna and Pfizer vials, with the SV40 sequence found only in the Pfizer vials. However, latent SV40 infections in a significant portion of the population could present the same SV40 risk to Moderna recipients. Even in the absence of chromosomal integration, the DNA plasmids could generate mRNA for the S-protein toxin and other harmful proteins for prolonged and unpredictable periods of time. Integration of foreign DNA into the human genome disrupts existing natural genetic sequences; this carries further risk of disease including cancer” [164]. Due to the lack of formal and transparent assessment by regulators, the experts also noted that it is currently impossible to provide informed consent for these products, as their complete risks remain undisclosed and not fully understood.

How did such dangerous, large-scale contamination escape the scrutiny of public health officials, and were the manufacturers aware of the issue? It is important to note that the process-related impurities were absent from the COVID-19 mRNA products used in the registrational trials. Virtually all doses used in those trials originated from “clinical batches” produced using what is known as Process 1 [1]. As a post-authorization emergency supply measure for global distribution, however, a method much more suitable for mass production known as Process 2 was devised utilizing bacterial plasmid DNA [165]. The Process 2 alterations include modifications to the DNA template employed for RNA transcription, changes in the purification phase, and adjustments in the manufacturing process of LNPs [165]. 

Notably, batches produced using Process 2 showed significantly reduced mRNA integrity [146,166]. According to the protocol amendment, each batch of the Pfizer product manufactured using Process 2 was administered to approximately 250 participants aged 16-55 years, with subsequent comparative analyses of immunogenicity and safety carried out on 250 randomly chosen recipients of Process 1 batches [165]. As of this writing, there are no publicly available analyses comparing the safety and reactogenicity of Process 1 and 2 batches.

Another relevant concern is the potential biological impact of replacing all the uridines in the RNA molecule with N1-methylpseudouridine. This strategy is regarded as a useful way to enhance protein expression as part of mRNA therapeutics [167]. This was also considered a breakthrough innovation, since the CureVac mRNA vaccine (CureVac N.V.. Tübingen, Germany), lacking this innovation, was less effective than the Pfizer and Moderna formulations [168]. The boost in effectiveness is likely because such an alteration retards the degradation process and thus causes the mRNA to last much longer. While N1-methylpseudouridine is a natural molecule, normally it is only present as a substitute for uridine in a small percentage of the uridines in a sequence. Still to be determined is what effect the massive introduction of N1-methylpseudouridine into the cell might have on its own synthesis of new mRNA molecules [169].

In a remarkable discovery, Mulroney et al. observed that the mRNA vaccines induced antibodies in mice to proteins that could be synthesized from the mRNA code if it were frameshifted by one nucleotide. This was not seen in cells challenged with just the S-protein or in mice vaccinated with the Astra-Zeneca vaccine (AstraZeneca plc, Cambridge, United Kingdom), which is a DNA-based vaccine [170]. They suggested that it was the N1-methylpseduouridylation that caused the frameshift. Such unintended, off-target proteins have, in Mulroney et al.’s terms, “huge potential to be harmful,” in part due to potential homology with human proteins that could, in turn, induce autoimmune disease [170-172]. Based on a query of the MedDRA code “Autoimmune disorder” in the Vaccine Adverse Events Reporting System (VAERS), there was an 803% increase in autoimmune disorders per million doses administered when comparing the administration of Influenza vaccines from 2018 to 2020 with COVID-19 vaccinations from 2021 to 2023 (Figure 5) [173]. This represents an immense safety signal. Such fundamental questions and concerns about the technology should have been addressed before the products were delivered to hundreds of millions of people [174].

**Figure 5:** VAERS reports of autoimmune disease per million doses of COVID-19 mRNA (2021-2023) compared to Influenza (2018-2020) vaccinations Based on a VAERS query (https://vaers.hhs.gov/) using the MedDRA code “Autoimmune disorder”, there was an 803% increase in reporting rate per million doses administered when comparing Influenza vaccines administered from 2018 through 2020 to COVID-19 mRNA injections administered from 2021 through 2023. Notably, the reports exclude individuals with a history of an autoimmune disorder. Image credit: Jessica Rose (coauthor), [173]

Mechanisms underlying AEs

A complete discussion of the biological mechanisms that may explain the various AEs of the COVID-19 vaccines is beyond the scope of this paper. We therefore refer readers to these papers [26,175-181]. The mechanisms of molecular mimicry, antigen cross-reactivity, pathogenic priming, viral reactivation, immune exhaustion, and other factors related to immune dysfunction all reinforce the biological plausibility for vaccine-induced pathogenesis of malignant and autoimmune diseases [26, 182-185]. Both SARS-CoV-2 and the mRNA vaccines can trigger immune dysfunction along with a host of pathophysiological effects, including chronic inflammation, thrombogenesis, prion-related dysregulation, and endotheliitis-related tissue damage [180].

The mRNA vaccines offer unique mechanisms of immune activation that are quite distinct from the response to a viral infection. These mechanisms help explain the AE profile of these gene-based products. The S-protein itself is arguably the most toxic protein produced by the virus [180]. The distribution of mRNA-LNP across a diverse array of tissues facilitates the expression of S-proteins on cell surfaces across multiple cell types [186]. This, in turn, renders the target tissues susceptible to T-cell-mediated attack and subsequent destruction [109-111]. Notably vulnerable are tissues such as cardiac muscle and neuronal tissues [80,144], both characterized by limited repair and regenerative capacity. Furthermore, vascular tissues show widespread targeting and assault throughout the body [180].

Other components of the vaccines contribute to complex, poorly understood, and unpredictable AEs. These components include the lipid nanoparticles, in particular the ionizable cationic lipids, the polyethylene glycol (PEG), and various process-related impurities such as the DNA plasmids (discussed in the preceding section) recently detected by independent researchers [151,186]. Ionizable cationic lipids are known to be toxic, inducing pro-apoptotic and pro-inflammatory cascades [187]. Yet they are an essential component of the vaccines, supporting the more prolific synthesis of abundant S-protein from the mRNA.

More than three decades ago, researchers were aware of the unusual potential for synthetic cationic lipid nanoparticles to form amphiphilic aggregates, disrupt the cell membrane, induce an inflammatory response, and suppress immune function [188]. In fact, there is growing interest in an emerging new theory for immune function that can explain immune activation in the absence of overt infection. Seminal research by Matzinger and her immunogenetics research team at the US National Institute of Allergy and Infectious Diseases has pioneered the concept that immune responses are primarily driven by the need to defend against what is dangerous instead of what is foreign [189].

PEG, one of the primary adjuvant components of the COVID-19 mRNA vaccines, is believed to be a major factor in vaccine-induced anaphylactic shock, a well-established potential immediate SAE in susceptible individuals [190]. Conjugation of PEG to the nanoparticles increases its immunogenicity, causing complement activation and a subsequent acute and life-threatening reaction [191]. Furthermore, the combination of PEG with the vaccine-generated S-protein may contribute to sudden-onset pituitary disorders (pituitary apoplexy, with transition to acute hypophysitis) occurring within a week of COVID-19 vaccination [192,193]. Taieb and colleagues postulate that these vaccine components could trigger a systemic inflammatory response and circulatory problems associated with vaccine-induced thrombotic thrombocytopenia (VITT), resulting in pituitary hemorrhage or infarction [192]. Because the symptoms of pituitary apoplexy include headache, vertigo, fever, and myalgia (all common vaccine adverse reactions), the authors suspect that the actual rate of post-vaccine pituitary disorders is much higher than what has been typically recorded. In a Taiwan study, the rate of post-vaccination vertigo/dizziness appeared to be substantially higher among recipients of Moderna’s mRNA-1273 compared to Pfizer’s BNT162b2, with the median time to the onset of vertigo/dizziness being 12 days and six days, respectively [194].

There is a large and growing literature describing the remarkable toxic effects of the S-protein. Its persistence for up to 30 days following vaccination is of great concern [195]. The S-protein causes an acute inflammatory response, through activation of the NF-κB signaling pathway [196]. It has been shown to induce senescence in endothelial cells, and this likely contributes to the diverse vascular-related AEs [197]. Of great concern is its amyloidogenic potential, which may play a significant role in the broad spectrum of neurological symptoms [198].

Following COVID-19 mRNA vaccination, particularly in young adults, many studies have found increased risks of myocarditis and cardiac arrhythmias, in some cases leading to sudden death [57,60,140,149,199-202]. The S-protein persists in circulation in young adults who developed myocarditis post vaccination, but not in vaccinated individuals who did not develop myocarditis [202]. Vaccine mRNA was isolated in the human heart at autopsy out to 30 days [195]. Direct cardiotoxicity of the Pfizer and Moderna mRNA vaccines on rat cardiomyocytes has been documented 48 hours after the injection [80]. S-protein and active inflammation were observed upon biopsy in young individuals hospitalized with COVID-19 vaccine myocarditis [203]. Cadegiani has proposed that a surge of adrenalin is a major precipitating factor in triggering cardiac arrest in young persons who suffer cardiac arrest in the setting of clinical or subclinical myocarditis [204]. An additional cardiotoxic mechanism may involve downregulation of angiotensin-converting enzyme 2 (ACE2) receptor expression following its binding to the S-protein. This can lead to unopposed ACE expression, increased angiotensin-2 levels, inflammation, and, ultimately, apoptosis [201]. Elevated angiotensin-2 causes inflammation and oxidative stress, which are major contributing factors in the progression of cardiomyopathy [205].

Generic immune suppression emerging after repeated booster injections poses another major concern. T-cell exhaustion refers to an immunologic condition in which CD8+ T cells show a progressive loss of cytokine production and cytotoxic potential [206]. Such dysfunction is known to occur in conditions such as chronic infections, cancer, and autoimmune diseases [207,208]. After three and four doses of the COVID-19 mRNA vaccine, researchers observed a diminished T-cell response against the S-protein, associated with a class switch to IgG4 [209]. Not only does IgG4 not protect from infection, but it actively blocks other IgGs to suppress their action, leading to immunosuppression [210]. Notably, a reduced T-cell response against SARS-CoV-2 was observed one month after receiving the third and fourth doses [211]. Such T-cell exhaustion in the wake of multiple COVID-19 mRNA inoculations could help explain the findings from studies showing increased rates of COVID-19 with increased frequency of boosters [99,100].

Loacker et al. demonstrated a significant increase in the expression of programmed death ligand 1 (PD-L1) on the surface of immune cells, measured two days following the second mRNA injection [212]. The binding of PD-L1 to PD-1 found on cancer cells restricts the ability of T cells to eliminate cancer cells, thereby facilitating tumor immune evasion [213]. Elevated levels of PD-L1 on immune cells may predispose cancer patients to unfavorable outcomes, and treatments that target PD-L1 suppression (anti-PD1 blockade) are gaining traction as viable therapeutic options [214]. Rapid progression of various lymphomas has been linked to COVID-19 mRNA vaccinations [215-218], and elevated PD-L1 may play a role in this context.

Other factors related to the oncogenic and tumor-hyperprogressive potential of the COVID-19 vaccines have become a focus of intensive inquiry. A recent review by Angues and Bustos explores the hypothetical capacity of COVID-19 vaccines to activate biological mechanisms that may collectively create a microenvironment conducive to cancer progression, either accelerating existing macroscopic disease or awakening dormant micrometastases [219]. These mechanisms relate primarily to the pro-inflammatory effects of the S-protein and LNPs, disruptions in the body’s ability to generate type I interferon, and disturbances in the regulation of cellular microRNAs caused by the altered structure of mRNA within the vaccines [219]. Additionally, the COVID-19 mRNA vaccines elicit elevated concentrations of interleukin-17 (IL-17) and upregulation of Th17, thereby disrupting Th1-Th2 immunity, escalating the chronic inflammatory condition of cancer patients, and further amplifying tumor growth and progression [220-222].

Immunologic basis for vaccine inefficacy

The biomedical purpose of the COVID-19 mRNA vaccination is basically twofold: (1) to leverage the body’s immune defenses against infection by SARS-CoV-2, and (2) to reduce the risk of severe disease and its consequences. Following intramuscular injection with the mRNA product, the S-protein-encoding mRNA is delivered via LNPs to human cells that generate S-proteins and/or related antigens that resemble those present on the surface of the coronavirus [25]. These antigens then stimulate the production of memory T-cells and B-cells, with the latter subsequently producing antibodies that bind to specific epitopes of the virus. Consequently, if a vaccinated individual encounters SARS-CoV-2, their immune system will mount a robust adaptive immune response in the short term, theoretically reducing the severity of the infection. This reduction in COVID-19 symptoms represents the intended clinical benefit of these biologicals.

The above explanation, however, connotes an immunologic disconnect between the systemic effects of the COVID-19 vaccination and the protection naturally afforded by lung mucosal immunity. SARS-CoV-2 is primarily an airborne virus that enters the human body via the upper respiratory tract. Thus, the immune system’s first encounter with the pathogen usually occurs in the nasal passages and tonsils, inducing the production of secretory IgA antibodies in saliva, nasal fluid, tears, and other secretions within just four days of the initial exposure [223]. The virus is then successfully confined to the upper respiratory tract, resulting in either asymptomatic infection or mild symptoms such as a cough or sneeze [223]. The combination of secretory IgA and activated tissue-resident T-cells in mucosal areas can halt the infection altogether, rather than just limiting the infection and curbing disease symptoms [224]. Moreover, based on studies of SARS-CoV (the presumed predecessor to SARS-CoV-2), the cellular immunity that accompanies the initial respiratory infection may persist for up to 17 years, even without a detectable humoral component [225]. In research involving human participants who consented to exposure to the H1N1 flu virus, pre-existing mucosal IgA provided better protection against severe illness than systemic IgG [226], suggesting that high circulating IgG titers might not correlate with robust protection. The lung mucosa produces an array of innate immune factors (e.g., complement, proteases, lactoferrin, and antimicrobial peptides) that work in synchrony with secretory antibodies (sIgA and sIgM) to limit the entry of foreign microbes and particles [227]. During infection, neutrophils are the predominant responders, releasing IL-8 and elastase to enhance the recruitment of natural killer cells, monocytes, and eosinophils from the circulation [227].

Given this immunological context, it is reasonable to surmise that the natural mucosal immunity against SARS-CoV-2 and other respiratory viruses may typically lead to more comprehensive, long-lasting protection compared to the systemic immune responses elicited by the COVID-19 vaccinations. Whereas SARS-CoV-2 infection induces both mucosal and systemic immune responses, the COVID-19 mRNA vaccines, as currently administered, are ineffectual in terms of inducing mucosal immunity [227,228]. The presumed benefits of vaccine-induced immunity are further counterbalanced by the SAE risks discussed previously. It cannot be overemphasized that these risks pertain to the entire population, the vast majority of whom have the capacity to eliminate SARS-CoV-2 without succumbing to severe morbidity or premature death.

When federal officials said the COVID-19 mRNA vaccines were “safe and effective”, they often added that the products were “95% effective against the infection”. Nonetheless, later studies showed that any protective benefit was short-lived, with immunity waning after only a few months [229,230]. This waning effect becomes more pronounced with successive boosters [231]. There is a logical explanation for this phenomenon. First, due to viral evolution, SARS-CoV-2 variants are constantly mutating, and numerous mutations have occurred in the S-protein, the intended target for neutralizing antibodies. These mutations, mostly concentrated in the vicinity of the receptor-binding domain (RBD), create constant opportunities for the generation of new escape variants (i.e., those that evade neutralizing antibodies), thus enabling immune evasion in subsequent vaccinations. Second, confrontation with novel antigens on escape variants is associated with “original antigenic sin”, the production of cross-reactive antibodies that may not be effective against the new antigen or pathogen due to prior exposure to predecessor strains [232,233]. Although cross-neutralization is a rare event, cross-reactivity in antibody binding to S-protein is common in the context of SARS-CoV-2 infection [234]. Additionally, other research indicates a degree of cross-reactivity between seasonal coronaviruses and SARS-CoV-2 [235].

When the immune system becomes entrained on preexisting SARS-CoV-2 variants, there is a progressive narrowing of the antibody response to the current, prevailing variants. This imprinting phenomenon has been demonstrated with respect to both natural infection and COVID-19 vaccination [236]. A 2021 pilot study found robust increases in humoral responses in SARS-CoV-2-naïve individuals following each dose of BNT162b2, whereas previously infected individuals showed strong humoral responses to the first dose of the mRNA injection but muted responses to the second dose [237]. Immune imprinting was also identified as the underlying factor contributing to the unanticipated decrease in the effectiveness of the bivalent COVID-19 vaccines since the “immune systems of people immunized with the bivalent vaccine, all of whom had previously been vaccinated, were primed to respond to the ancestral strain of SARS-CoV-2” [238].

At least part of the immunologic basis for COVID-19 vaccine failure can be summarized as follows. SARS-CoV-2’s S-protein binds to the ACE2 receptor, creating a scenario wherein strong selective immune pressure prompts the S gene to mutate and develop viral escape mechanisms. Since the majority of SARS-CoV-2 vaccines are designed using the S-protein sequence from the initial Wuhan strain, these escape mutants can effectively evade the immune responses triggered by these vaccines. This leads to reduced effectiveness of all subsequent injections with mRNA products utilizing the original S-protein sequence [236,239,240]. Periodic COVID-19 mRNA inoculations may adversely impact viral ecology and encourage the ongoing emergence of immune escape variants (i.e., variants escaping the selective pressure via mutation) that ultimately render the vaccines ineffective. Such diminishing returns were observed in the Cleveland Clinic studies discussed earlier in this paper [99,100]. Additionally, ongoing boosters are likely to cause immune dysfunction, thereby diminishing antiviral and microbial protection while promoting autoimmune disease and accelerated cancer progression.

Given the ongoing genetic changes in SARS-CoV-2 driven by both natural viral evolution and vaccine-induced selective pressure on the immune system, it is likely that frequent COVID-19 mRNA vaccinations would need to be administered in the coming years to address new prevailing variants. However, the immune imprinting noted above could limit the ability to achieve robust protection and could potentially facilitate viral transmission even with population-wide vaccination [239]. Immune evasion by new or emerging SARS-CoV-2 variants in individuals vaccinated against former variants will continue indefinitely, due to antibody cross-reactivity and immune imprinting.

Somewhat ironically, then, the mRNA vaccines’ ability to perpetuate the emergence of new variants also tends to engender the perception among the general public that a new round of boosters is necessary. This, in turn, sets up an endless vaccine-escape variant cycle, a feedback loop whereby the actions taken to address the issue (more vaccinations) inadvertently contribute to ongoing inefficacy. Mutations in the viral S-protein provide resistance against antibody responses, and this selection process underlies the larger phenomenon in which new dominant variants are emerging [241-243]. Mass mRNA inoculations result in the natural selection of highly infectious immune-evading SARS coronavirus variants that successfully bypass vaccine-induced immunity, leading to a dramatic rise in the prevalence of these variants [108]. 

In summary, the large-scale emergence of dominant variants was an adaptive response to the selection pressure exerted by the mass vaccination campaign, a response further heightened in immunosuppressed individuals [244]. Importantly, the immune-escape mutants are developing primarily in vaccinated individuals, not in the unvaccinated [245,246][241,242]. Mechanisms underlying vaccine-induced immune dysfunction (see preceding section) contribute further to the inefficacy. The main factors involved in COVID-19 mRNA vaccine inefficacy are summarized in Figure 6 [247].

**Figure 6:** Factors contributing to COVID-19 mRNA vaccine inefficacy COVID-19 vaccines may lose efficacy in part by inducing SARS-CoV-2 mutations that lead to new immune escape variants, thus ultimately limiting vaccine-related protection against subsequent coronavirus infections. Periodic COVID-19 mRNA injections could elicit a diverse range of mechanisms associated with immune dysfunction (mostly due to subversion of innate immunity), resulting in a heightened risk of cancers, infections, and autoimmune disorders. Image Credit: Majumder and Razzaque, 2022 [247]; adapted with permission from authors.

Discussion

In this review, we consider alternate narratives based on a direct assessment of available data and published studies. By doing so, our intention is to foster transparency, trust, and informed decision-making, ensuring that the public’s legitimate questions concerning COVID-19 vaccine safety are addressed. This approach not only contributes to the ongoing discourse surrounding safety but also paves the way for the improvement in public health strategies going forward. The ethical implications of our inquiry relate to epidemiological inequities: whereas COVID-19 has primarily afflicted the immunosuppressed, elderly, and those with multiple comorbidities, the COVID-19 vaccinations have the potential to adversely impact people of all ages, not only frail elderly individuals (the most vulnerable sub-group) but also young and relatively healthy individuals, most of whom have a near-zero risk of serious consequences from COVID-19 [40]. When we consider the likelihood of more frequent SAEs resulting from interactions between COVID-19 mRNA vaccination and subsequent SARS-CoV-2 infections, it is important to bear in mind that the Omicron subvariant infections that have been dominant since early 2022 follow a mild course and are invariably non-lethal [248]. Moreover, whereas infections by their very nature are involuntary and accidental, the mRNA injections are a choice with potentially life-threatening repercussions.

The pivotal role of randomized placebo-controlled clinical trials in assessing the efficacy of vaccines and other interventions has long been recognized within the medical and public health communities. The value of well-designed controlled trials was highlighted in a report by the WHO Ad Hoc Expert Group on the Next Steps for COVID-19 Vaccine Evaluation published in January 2021 [249]. Ensuring the credibility of observed outcomes, particularly in the context of novel experimental drugs such as modified RNA-LNP products, entails a meticulous process of randomly assigning subjects meeting various criteria to either intervention or placebo groups. Randomization not only establishes a baseline for comparison but also facilitates the attribution of any differences in outcomes to the intervention itself. The placebo control minimizes the chances of erroneous conclusions about the intervention’s effects. Although invaluable as tools for detecting safety signals, national health surveillance databases such as VAERS and Yellow Card do not meet the rigorous standards set by controlled trials, further underscoring the necessity of this approach for the assessment of medical and public health interventions.

In retrospect, the most concerning revelation from the registrational trials that led to the EUA was not the apparent overstatement of 95% efficacy, but rather the indication within those trials that the vaccines carried a significant risk of SAEs and premature death, even among a relatively healthy group of participants. Based on the extended Pfizer trial findings, our person-years estimate yielded a 31% increase in overall mortality among vaccine recipients, a clear trend in the wrong direction. Moreover, the Fraiman et al. analysis showed a significant 36% higher risk of SAEs (including deaths and many life-threatening conditions) in the vaccine group for the Pfizer trial [50]. The Michels et al. analysis found a nearly four-fold increase in cardiovascular SAEs among subjects in the Pfizer trial who received the BNT162b2 injection compared to placebo, a fact never reported to the public at the time of the rollouts in December 2020 [54]. Notwithstanding these grave concerns, the Moderna product has shown even more frequent AEs when compared to its Pfizer counterpart [116-120,135]. Both mRNA products were linked with increased risks of ischemic stroke, brain hemorrhage, acute coronary syndrome, and other conditions known to reduce life expectancy.

Against this backdrop, and, in particular, given the high NNV (~52,000 vaccinations needed to prevent one COVID-19 death), the rationale behind the FDA’s decision to declare the COVID-19 mRNA vaccines “safe and effective” for worldwide distribution after only 20 weeks of observation seems dubious at best. Indeed, one might have expected the COVID-19 mRNA vaccines to have been withdrawn from the market following the Fraiman study’s revelation of one SAE in 800. The 1976 swine flu vaccine was pulled after being associated with Guillain-Barré Syndrome at a rate of approximately one in 100,000 [250]. The rotavirus vaccine Rotashield was withdrawn following reports of intussusception in one or two in 10,000 vaccinees [251]. In the case of the mRNA vaccines, Fraiman’s team reported their preliminary findings to both the FDA and EMA. Leaders from both agencies met with the team and provided feedback that resulted in a revised analysis [50]. Nonetheless, the regulators took no action afterward to warn the public and restrict access to the injections.

Along similar lines, the forensic analysis by Michels et al. exposed serious flaws in the methods used by the FDA, CDC, and NIH in the development and safety/efficacy evaluation of new pharmaceutical products [54]. The authors concluded that “the decision to approve the BNT162b2 mRNA vaccine by the US FDA and other international regulatory agencies was not an informed decision based on an unbiased, thorough, and transparent evaluation of the evidence intended to demonstrate that this vaccine met the criteria that it was a ‘safe and effective’ means of controlling the COVID-19 pandemic" [54]. Pfizer had an ethical responsibility to proactively disclose any new information that could impact the FDA’s decision-making process. Their failure to do so was factually misleading. Conversely, it is reasonable to expect that all participants in the VRBPAC meeting should have been aware that the trial’s mortality data from November 14, 2020, had become outdated. Remarkably, no VRBPAC members inquired about updates on AEs that transpired between the EUA data cutoff date (November 14, 2020) and the date of the meeting (December 10, 2020) [54].

According to a 393-page confidential document requested by the EMA and released in August 2022 [114], Pfizer had by that time documented approximately 1.6 million AEs covering nearly every organ system [114, 252,253]. One-third of the AEs were classified as serious. Among the many findings were 3,711 tumors, 264 categories of vascular disorders (73,542 cases total), over 100,000 blood and lymphatic disorders, 127,000 cardiac disorders (including 270 categories of heart damage in addition to myocarditis and pericarditis), 77,000 psychiatric disorders (including psychoses, depression, suicide and suicidal behaviors), and hundreds of categories of neurological disorders (696,508 cases total), many of which are considered very rare, a clear indication of grave hazards. These estimates offer a striking contrast with the official FDA document titled “Summary Basis for Regulatory Action” dated November 8, 2021, in which the review committee voted to approve the Pfizer-BioNTech product [56]. The report’s entire “Risk-Benefit Assessment” section consists of a single sentence: “Considering the data submitted to support the safety and effectiveness of COMIRNATY that have been presented and discussed in this document, as well as the seriousness of COVID-19, the Review Committee is in agreement that the risk/benefit balance for COMIRNATY is favorable and supports approval for use in individuals 16 years of age and older" [56].

International analyses of excess mortality indicate that COVID-19 vaccinations may have had serious largescale consequences. In a careful study of mass vaccinations throughout Europe in 2021-2022, Aarstad and Kvitastein analyzed the potential interplay between COVID-19 vaccination coverage in 2021 across Europe and subsequent monthly excess mortality through 2022 [254]. Utilizing a well-curated dataset encompassing 31 nations, the authors applied population-weighted analyses and found the following: (a) increases in ACM during the initial nine-month period of 2022 were positively correlated with increases in 2021 vaccination distribution; and (b) each percentage point increase in 2021 vaccination coverage was associated with a 0.105% increase (95%CI 0.075-0.134) in monthly mortality during 2022. An extensive, multi-country ecological analysis by Rancourt and colleagues estimated that COVID-19 vaccination resulted in 17 million excess deaths, with a global vaccine-dose fatality rate (vDFR) of 0.1257 ± 0.0035%, or approximately 0.1% [251]. Rancourt’s 180-page report showed that the COVID-19 vaccine rollouts were synchronously followed by peaks in all-cause mortality in many countries [255,256].

While most vaccinees have an extremely low risk of COVID-19 hospitalization and death, they face a relatively high risk of SAEs (one SAE for every 800 injections) following the COVID-19 mRNA vaccination [50]. This disturbing dichotomy is most pronounced in the context of the childhood immunization programs, although in fact all ages under 40 show near-zero IFRs. Pezzullo et al. calculated median IFRs of 0.0003% at 0-19 years, 0.002% at 20-29 years, and 0.011% at 30-39 years [40]. As noted earlier, death rates among children have been extremely low even in countries showing excess mortality during the pandemic [43], and allowing children to attend school freely, as occurred in Sweden, resulted in zero COVID-19 deaths among this younger age group [44]. Given this very low risk to children, we must reject the policy of administering an experimental vaccine to these age groups. Against the (then dominant) Omicron subvariant, BA.5, the bivalent mRNA vaccines were only tested in eight mice, never in humans [257]. Following this authorization, noted vaccinologist Paul Offit, a member of the VRBPAC, wrote: “We should stop trying to prevent all symptomatic infections in healthy, young people by boosting them with vaccines containing mRNA from strains that might disappear a few months later" [237]. Based on the best available evidence, the potential risks of these mRNA inoculations have consistently outweighed the benefits for younger generations [258,259]. Consideration of a harm-to-reward calculus weighs heavily on factors like lymphomas [215-218] and heart damage [57-63] in these younger age groups. With regard to cardiac risks, prospective studies with careful assessments of potential myocardial damage have found that the risk of ambulatory young individuals developing myocarditis is about 2.5% (2500 per 100,000 recipients) for either BNT162b2 or mRNA-1273 following the second or third injections [260,261]. The 2.2% myocarditis risk in adolescent teens following the COVID-19 mRNA injection is approximately 37 times the risk associated with SARS-CoV-2 infection (0.06%) in that same age group [260,262]. Given these estimates, there is no valid reason for vaccinating this age group.

Figure 7 shows a graph based on myocarditis reports in VAERS Domestic Data as of September 29, 2023, which offers an indication of the gravity of this situation. All myocarditis reports are plotted according to age and dose (dose 1 (pink), dose 2 (green), and dose 3 (blue)). After dose two, there was a five-fold increase in myocarditis cases among 15-year-old males. Regardless of age, myocarditis cases were more frequent following dose two, which is suggestive of a causal link between myocarditis and the COVID-19 mRNA inoculations. The data depicted in the chart are further reinforced by a recent disproportionality analysis of VAERS data showing a statistically significant association between cardiovascular events and COVID-19 vaccinations [263].

**Figure 7:** Myocarditis reports in VAERS Domestic Data as of September 29, 2023, plotted by age and dose Dose 1: pink, Dose 2: green, Dose 3: blue Data indicates a five-fold rise in myocarditis cases after the second COVID-19 shot for 15-year-old males, and overall, second doses were linked to more myocarditis cases [263]. VAERS: Vaccine Adverse Event Reporting System; COVID-19: coronavirus disease 2019 Image Credit: Jessica Rose (coauthor).

The adverse impacts on younger segments of the population were also reflected by the extraordinary reports from US life insurance companies for the latter half of 2021. According to the Group Life survey data, during Q3 and Q4 of 2021, the general US population experienced a 32% increase in mortality compared to 40% in the Group Life count (8% difference) [264]. Group Life Policyholders are well-employed, young, and generally healthy adults, previously dying at about one-third the rate of the US population, based on a 2016 Society of Actuaries (SOA) analysis [264]. Thus the mortality observed among the Group Life cohort in 2021 represents an inversion of previous trends. The excess deaths in the Group Life data were determined by comparing average death rates in the Group Life data from the 2017-2019 baseline, adjusted for seasonality and combined with CDC data. Between Q2 and Q3, the beginning of the second US vaccination rollout, the SOA analysis showed a 36% increase in excess mortality for ages 25-34, a 50% increase for the 35-44 age group, and a 52% increase for the 45-54 age group [264]. These numbers represent colossal and unprecedented increases in excess mortality for the 25-54 age range, with an average increase of 46% (though averaging the percentages tends to mask the severity of the impact on specific age cohorts) [264].

As mentioned above, these were younger, healthier adults, and thus it is illogical to suggest that COVID-19 had any substantial influence on mortality, especially given the extremely low IFR associated with the younger age brackets. Indeed, according to the most recent Group Life report, the excess mortality in each of the age groups applied only to “non-COVID-19” deaths; there was no excess mortality directly attributed to COVID-19 [264]. Importantly, the surge in excess mortality among the 25-54 age group was also temporally associated with the introduction of US vaccine mandates among military and hospital personnel from the summer into the fall of 2021 [265]. From March 2021 to February 2022, there were approximately 61,000 excess deaths among Americans under age 40, equivalent to all US servicemen lives lost during the Vietnam War [266]. This tragedy was never reported by any of the major US news media.

The health-related repercussions of these vaccine-related heart risks have been manifesting on the public stage since 2021. Prior to that year, the average annual number of cardiac arrests on the field for professional athletes in Europe was 29; this number has risen to 283 per year, an approximately 10-fold increase, based on the annualized rate of cardiac arrests following the vaccination program’s inception for active players aged 35 [267]. Two-thirds of the players were not resuscitated [267]. Recent research suggests there may be a genetic basis (SCN5A variants) for sudden deaths occurring within seven days of COVID-19 vaccination, regardless of vaccine type, number of doses, and underlying diseases [268]. By identifying genetic risk factors (e.g., MTHFR polymorphisms) before receiving the COVID-19 vaccine, the risks of venous thromboembolism and other vaccine-related vascular injuries can be more effectively addressed [269,270].

The World Council for Health has demanded an immediate moratorium on these novel products [164], due in part to the issue of extensive DNA contamination. On a precautionary basis, we agree with recommendations for the immediate removal of the COVID-19 vaccines from the childhood immunization schedule along with the suspension of boosters and a full investigation of the vaccine industry’s and regulatory agencies’ misconduct regarding safety assessments and data from the founding trials. It is unethical and unconscionable to administer an experimental vaccine to a child who has a near-zero risk of dying from COVID-19 (IFR, 0.0003%) but a well-established 2.2% risk of permanent heart damage based on the best prospective data available. Additional risks for these otherwise healthy young individuals include seizures, cancers, autoimmune disorders, and numerous other life-stealing conditions post vaccination.

Another relevant aspect of this unfolding tragedy is the untold story of reduced life expectancy. In many developed countries, the main causes of reduced life expectancy (smoking, obesity, opioid overdose, homicides, suicides, and infant mortality) are the primary causes of premature death on a population scale [271]. Nevertheless, it is also clear that several risks associated with COVID-19 vaccinations may translate into premature death in the long term. Among the poor, untreated bacterial pneumonia is a major cause of reduced life expectancy and may be further exacerbated by COVID-19 vaccination [272]. Strokes and myocarditis associated with COVID-19 vaccinations may cause premature death years after the initial event. A longitudinal study of stroke patients found that fewer than 28 days after a stroke, the risk for death was 28%; this increased to 41% at one year and 60% at five years [273]. Undiagnosed heart and clotting problems can persist asymptomatically for years. Multiple autopsy studies provide definitive evidence of serious post-injection damage to the heart, including sudden cardiac arrest and sudden death, all associated with the COVID-19 mRNA vaccines [140]. In adolescent males, however, myocarditis can have a mild outward clinical appearance yet result in severe cardiac fibrosis (scarring), with permanent damage to the heart muscle [274,275]. Such damage can eventually lead to congestive heart failure and death many years later [276]. The registrational trials were insufficient for detecting these long-range hazards, most of which only became evident after 2.5 years of follow-up observation and over a billion mRNA injections.

Also germane to this discussion is the medically intractable phenomenon known as “long COVID”. After the acute phase of a SARS-CoV-2 infection, some individuals experience persistent symptoms like fatigue, brain fog, muscle pain, breathing difficulties, tingling extremities, and chest and throat discomfort for extended periods. This has come to be known as post-acute COVID-19 syndrome (PACS), a multifactorial, multisystemic condition encompassing dysautonomia, encephalitis, chronic fatigue syndrome, immune dysfunction, cardiovascular and clotting abnormalities, and impacts on multiple organ systems [277]. Specific types of PACS can be defined based on the presentation of symptoms [278,279]. Not surprisingly, because of the common denominator between infection and mRNA inoculation (the S-protein), COVID-19 vaccination produces long-term symptoms that share many features with PACS [280,281]. The condition may be triggered by an immune overreaction to the vaccine-generated S-protein [282], which has been shown to persist at least six months after the injection [283]. Vaccine-associated S-protein has been found in PACS patients [284,285]. Diexer et al. observed that 70% of PACS cases occurred in individuals who had received full COVID-19 vaccination, indicating that the injections may exacerbate PACS in most cases [286]. The group with the lowest risk of PACS was the unvaccinated individuals who contracted Omicron as their first infection. Thus, contrary to popular beliefs and media messaging, vaccinated individuals may experience more severe long-term outcomes of COVID-19 compared to the unvaccinated. Several new syndromes associated with the mRNA inoculations have been introduced that encompass conditions very similar to PACS: post-COVID-19 vaccination syndrome (PCVS), acute COVID-19 vaccination syndrome (ACVS), and post-acute COVID-19 vaccination syndrome (PACVS) [287]. It has been proposed that the forthcoming version of the International Classification of Diseases (ICD) diagnostic codes should incorporate a new code specifically for “post-COVID-19 vaccination condition, unspecified" [287].

In addition to addressing the complex, post-COVID-19 vaccine-related conditions alluded to above, it is our bioethical imperative to carefully consider other consequences of ongoing, repeated boosters. Broadly speaking, these consequences may be divided into two categories: (1) diminishing returns following the injections due to various immune-suppressive effects along with extrinsic selective pressures that ultimately accelerate viral evolution and resistance; and (2) SAEs, notably the profound suffering and premature death resulting primarily from autoimmune, neurological, malignant, and cardiovascular disorders. Consideration of both the potential immunological impacts of repeated booster doses on viral evolution and resistance alongside the risks of premature death and other SAEs is crucial for a comprehensive risk-benefit assessment of the mRNA COVID-19 vaccinations, ensuring informed public health decisions.

Based on the research presented in this narrative review, the global COVID-19 vaccination campaign should be regarded as a grave medical error. Medical errors represent a substantial threat to personal and public safety and have long constituted a leading cause of death [288-290]. Misguided political and regulatory decisions were made at the highest levels and may have been heavily influenced by financial incentives. Government agencies should have considered all reasonable treatment alternatives and deflected pressures away from the medical-pharmaceutical industry rather than allowing population-wide distribution of experimental genetic vaccines. Had the FDA recognized the nearly four-fold increase in cardiac SAEs (including deaths) subsequently identified in the Pfizer trial’s vaccine group [54], it is doubtful that the EUA would have transpired in December 2020. An in-depth investigation of the COVID-19 vaccine’s long-term safety profile is now urgently needed. Despite the many striking revelations discussed in this review, most developed countries continue to advocate the ongoing adoption of COVID-19 mRNA boosters for the entire eligible population. US federal agencies still emphasize the safety of the vaccines in reducing severe illness and deaths caused by the coronavirus, despite the absence of any randomized, double-blind, placebo-controlled trials to support such claims. This reflects a bewildering disconnect between evidence-based scientific thinking and public health policy.

## Conclusions

Careful, objective evaluation of COVID-19 mRNA product safety is crucial for upholding ethical standards and evidence-informed decision-making. Our narrative review concerning the registrational trials and the EUA’s aftermath offers evidence-informed insights into how these genetic vaccines were able to enter the market. In the context of the two pivotal trials, safety was never assessed in a manner commensurate with previously established scientific standards either for vaccines or for GTPs, the more accurate classification of these products. Many key trial findings were either misreported or omitted entirely from published reports. The usual safety testing protocols and toxicology requirements were bypassed by the FDA and vaccine manufacturers, and the premature termination of both trials obviated any unbiased assessment of potential SAEs due to an insufficient timeframe for proper trial evaluation. It was only after the EUA that the serious biological consequences of rushing the trials became evident, with numerous cardiovascular, neurological, reproductive, hematological, malignant, and autoimmune SAEs identified and published in the peer-reviewed medical literature. Moreover, the COVID-19 mRNA vaccines produced via Process 1 and evaluated in the trials were not the same products eventually distributed worldwide; all of the COVID-19 mRNA products released to the public were produced via Process 2 and have been shown to have varying degrees of DNA contamination. The failure of regulatory authorities to heretofore disclose process-related impurities (e.g., SV40) has further increased concerns regarding safety and quality control oversight of mRNA vaccine manufacturing processes.

Since early 2021, excess deaths, cardiac events, strokes, and other SAEs have often been wrongly ascribed to COVID-19 rather than to the COVID-19 mRNA vaccinations. Misattribution of SAEs to COVID-19 often may be due to the amplification of adverse effects when mRNA injections are followed by SARS-CoV-2 subvariant infection. Injuries from the mRNA products overlap with both PACS and severe acute COVID-19 illness, often obscuring the vaccines’ etiologic contributions. Multiple booster injections appear to cause immune dysfunction, thereby paradoxically contributing to heightened susceptibility to COVID-19 infections with successive doses. For the vast majority of adults under the age of 50, the perceived benefits of the mRNA boosters are profoundly outweighed by their potential disabling and life-threatening harms. Potential harms to older adults appear to be excessive as well. Given the well-documented SAEs and unacceptable harm-to-reward ratio, we urge governments to endorse and enforce a global moratorium on these modified mRNA products until all relevant questions pertaining to causality, residual DNA, and aberrant protein production are answered.

## Appendices

Appendix 1

Appendix 2

Regarding potential harms, assuming 30% false-positive reports and a moderate under-reporting factor of 21, we calculate a risk of 27 deaths per 100,000 doses of BNT162b2. Thus, applying these reasonable assumptions, the estimated harms of the COVID-19 mRNA injectables outweigh the rewards by nearly 14-fold.  

This mortality analysis combines two groupings of data, the first reflecting benefits, and the second reflecting harms. The first data grouping assumes one is saving lives by using the vaccine to prevent severe COVID-19 symptoms and hospitalization, based on the Pfizer and Moderna founding RCTs. The second grouping utilizes data from injury-reported databases, specifically the UK Yellow Card data as obtained by Norman Fenton and colleagues [291]. The Fenton data is “per dose” so is effectively doubled to a “course” consisting of two injections. The Excel (Microsoft Corporation, Redmond, Washington, United States) formula is based on the rules of joint probability: P(A & B) = P(A) + P(B) - P(A)*P(B) (assuming two events are independent). It turns out that: P(A)*P(B) is small, so in effect, it is P(A) + P(B), which if A=B is 2*P(A).

Benefits/Rewards

Calculations for the number of lives saved per 100K vaccinations, based on most generous assumptions are as follows: Assuming NNV of 119 and IFR of 0.23%, about ~52,000 vaccinations would be needed to prevent one death. Upper limit of lives saved per is 10,000*1/52,000 =  0.19 or ~0.2 or 1/5 of a life is saved for every 10,000 courses of the mRNA vaccine. Thus, for Pfizer mRNA vaccination, ~2  lives were saved from COVID-19 for every 100,000 courses of the vaccine.

Sources informing the numbers used in this estimate:  NNV to prevent a case is 119, based on data from Olliaro et al., 2021 [66], and assuming the infection-fatality ratio of COVID-19 is generously estimated at 0.23%, based on 2021 WHO data from Ioannidis: https://apps.who.int/iris/handle/10665/340124

Estimates of IFR are based on meta-analysis and NNT obtained from the Phase 3 Pfizer trial.  Given evidence of RCT fraud, this estimate should be viewed as an upper bound; the true value is likely much lower (i.e., even fewer lives saved).

Risks/Harm

Lives lost per 100,000 vaccinations-calculations based on the most conservative assumptions (URF=10): Fenton calculates 68 deaths/1,000,000 doses = 12.8 deaths per 100,000 per primary course of Pfizer, or just under 13 deaths from serious adverse events per 100,000 for each primary course of the Pfizer vaccine. Comparing AEs to potential benefits, we calculate an excess death risk of 12.8 - 2 = ~11 deaths per 100,000 doses. Thus, comparing the benefits to harms, at least 5 times more lives are lost than saved by the full course of Pfizer mRNA vaccinations.

Notes on the estimate:  Fenton number of 12.8 indicates an excess death risk of 12.8 - 2 = ~11/100,000 comparing the adverse effects to potential benefits. Our estimate is therefore alleging about one excess death per 9,000 Pfizer courses, which seems quite plausible. This is also in line with officially reported all-cause deaths in the Pfizer trial being 15 vaccinated and 14 in unvaccinated, which is a ~7% increase, although obviously not statistically significant. If there is one excess death per 9,000 jabs, a difference of ~2 deaths in 20,000 subjects/arm in the Phase-3 trial (one observed, but could be more) would be expected.  Finally, a higher URF (e.g., 21, based on Rancourt data), would yield a higher estimate

Pfizer trial data, applying the same Fenton calculation sequence and 30% false-positive reports, with a moderately conservative URF of 21: (i) Lives saved per 100,000 vaccinated (by preventing one COVID-19 death): NNV to prevent one COVID-19 case = 59,574 (95% CI 51,118-71,381). Lives saved per 100,000 vaccinated = 1.7 (95% CI 1.4-2.0); (ii) Lives lost per million: Net excess deaths per primary Pfizer course: 3,705 (95% CI 3,667-3,744). Excess death risk of 27 deaths (95% CI 26.7-27.3) per 100,000 doses of Pfizer’s COVID-19 mRNA vaccine.

Moderna trial data, applying the same Fenton calculation sequence and 30% false-positive reports, but with a moderately conservative URF of 21: (i) Lives saved per 100,000 vaccinations (by preventing one COVID-19 death): NNV to prevent one COVID-19 case = 25,394 (95% CI 22,434-29,254). Lives saved per 100,000 vaccinated (by preventing one COVID-19 death) = 3.9 (95% CI 3.4-4.5); (ii) Lives lost per 100,000 vaccinations (by preventing one COVID-19 death): Net excess deaths per primary Moderna course = 9,292 (95% CI 8,864-9,764). Excess death risk of 10.8 deaths (95% CI 10.2-11.3)  per 100,000 Moderna vaccine courses. 

Interpretation/context:  There are three important numbers to consider in these calculations: net mortality, NNV, and net excess deaths per primary course. Net mortality is the overall mortality, including deaths caused by the vaccines as well as other cause of death that could be biologically plausible given the population.  In this case, however, the population is relatively healthy and “low risk” in terms of COVID-19-related mortality (relatively healthy population with no comorbid diseases at baseline), and thus any disproportionate increase in overall mortality must logically be linked with the vaccination.

The epidemiological meaning of “net excess deaths per primary (Pfizer or Moderna) course” (NEDPC) number is the net cumulative incidence of increased death expected after vaccination, within about three months of the vaccine. In our calculation, the NEDPC number is the reciprocal of the net mortality. The interpretation is in the context of the calculation, i.e., benefits versus harms, with fairly conservative assumptions made on the harm side (false-positive reports and under-reporting assumptions).

Based on the founding clinical trial timeframes, we assume that three months is the period of time in which the vaccine would either incur benefit in terms of lives saved (related to the duration of trial and/or immunity) or incur harm, as in serious adverse events related to the vaccination. In real-world observational studies, longer timeframes would likely reveal other serious adverse effects that could result in premature death.

We also assume a 30% false positive rate (very conservative) and differing underreporting factors (URFs) of 10 and 21. The underreporting range is 10-100, with the upper end based on Harvard data of Lazarus et al. [292]. Thus, the URF of 10 may be deemed extremely conservative, and the URF of 21 is modestly conservative. 

Calculation of the NNV is dependent on COVID-19 prevalence, and for this, we rely on the WHO website’s seroprevalence study by Ioannidis et al. [293]. Due to our use of the injury database data, the hierarchy of evidence would be considered lower than for the analyses from the papers of Fraiman et al. [50] and Classen [49], which relied only on RCT evidence.

All of our “harm data” is from the UK’s Yellow Card data set, which is stratified by vaccine in Fenton's analysis [291]. While this information comes from the UK population, the trials were principally conducted in North America; nevertheless, it is unlikely that the adverse event rates would be different between the two populations.
